# Fractional-Order Boosted Jellyfish Search Optimizer with Gaussian Mutation for Income Forecast of Rural Resident

**DOI:** 10.1155/2022/3343505

**Published:** 2022-06-13

**Authors:** Yang Lei, Lingyun Fan, Juntao Yang, Wenhu Si

**Affiliations:** ^1^School of Public Administration, Northwest University, Xi'an 710127, China; ^2^School of Architecture and Urban Planning, Suzhou University of Science and Technology, Suzhou 215011, China; ^3^Academy of Architecture, Chang'an University, Xi'an 710061, China

## Abstract

The disposable income of residents can reflect the living standard of people in the area. For government departments, it is necessary to master the trend of rural resident income to formulate corresponding policies benefiting farmers. Thus, this paper proposes a grey model with an improved jellyfish search optimizer to predict the rural resident income in Shaanxi Province. Firstly, by applying fractional-order modified strategy and Gaussian mutation mechanism to the original algorithm, the proposed algorithm shows better performance in solving accuracy, stability, and convergence acceleration when compared with different classical methods on cec2017 and cec2019 test functions. Then, based on the fractional time-delayed grey model, a discrete fractional time-delayed grey model with triangular residual correction (TDFTDGM) is proposed by replacing the derivative with a first-order difference and introducing the triangular residual correction functions. Finally, the improved jellyfish search optimizer is used to explore the optimal order of the TDFTDGM model. The all-around performance of the forecast model is incomparable to additional grey models compared on four measure criteria, which means it is a practical approach for long-term prediction with small samples. Moreover, the forecast data of rural resident income in Shaanxi Province from 2021 to 2025 are given for reference.

## 1. Introduction

Agriculture, rural areas, and farmers are important issues for the long-term stability of the country in China [1]. In addition, the income of rural residents is a key index, which reflects the living standard of people in rural areas and the economic development of rural farmers [2]. Only by understanding the trend of rural residents' income, the government is able to formulate a series of policies to improve the income of rural residents [3]. However, there are only a few empirical studies on income prediction in the current literature. It is because that it is highly difficult and time-consuming to get exact information about the disposable income of a region in a long period [4]. Meanwhile, due to the income being affected by policies, climate, and other uncertainty factors, it is a challenging task to predict the income accurately [5].

Though the forecasting models for resident income are scarce, there are many forecasting approaches for other areas. For example, Maaouane et al. used the multiple linear regression method to predict the industry energy demand in Morocco [6]. Radial neural network is also a popular tool, which was used for energy consumption forecasting and wind speed forecasting in [7, 8], respectively. The authors in [9, 10] used the ARIMA model to the daily production prediction of wells in Sulige and to forecast the rural population in China from 1970 to 2015. Although these approaches can complete the task of data prediction according to different features, there are some defects. A tremendous amount of sample data is required, which means the above methods are not suitable for problems with a small sample [11]. As a choice, the grey forecasting algorithm solves the prediction problem of a small sample data set.

The grey model (GM) is an effective forecast approach with microscopic samples, which was proposed in 1982 [12]. It has the benefits of simple calculation, heightened precision, and wide application. As scholars have a deeper understanding of GM, some enhanced models were presented to enhance the accuracy. The classic grey model (GM) is mixed with the trigonometric residual modification strategy. Zhou et al. proposed a novel trigonometric grey prediction approach (TRGM) to forecast electricity needs and obtain effective results [13]. Then, in [14], an unknown discrete grey forecasting model called the DGM was designed. It showed outstanding performance in predicting the long-term developing tendency of an information series. Meanwhile, Wu et al. proposed a novel nonlinear grey Bernoulli model with fractional-order accumulation, shortened as the FANGBM model in 2019 [15]. This model was used to predict increase trend of the future China's renewable consumption. Though the curtain-raiser of fractional-order collection has created meaningful contributions to forecasting methods, some issues may also be mistaken as they do not consider the time-delayed effect. Thus, the authors in [16] introduce a new fractional grey model, called the fractional delay grey model (FTDGM). We design a novel grey model to obtain better-predicted results considering the significance of the discrete model and trigonometric residual modification technique.

Moreover, there is a parameter to be determined in the fractional grey model, the fractional order. Then, how to choose the most suitable parameters becomes another thorny problem. The authors in [16] provided a practical solution, which applied a metaheuristic algorithm to select parameters.

Metaheuristic methods have been grown rapidly in current years and show outstanding performance in solving continuous, discrete, or nonlinear optimizations problems [17, 18]. Generally, metaheuristic algorithms can be categorized into four varieties, swarm intelligence (SI) algorithms, evolutionary algorithms (EAs), physics-based algorithms (PhAs), and human-based algorithms [19]. The cooperative and hunting behavior of social animals in nature inspire SI algorithms. Particle swarm optimization (PSO) is the most classical one, which has been employed to solve different problems [20]. With the exploration of animal habits in recent years, lots of SI algorithms have emerged. In 2015, Wang et al. proposed the monarch butterfly optimization (MBO) algorithm by simplifying and idealizing the migration of monarch butterflies [21]. After being compared with other algorithms on thirty-eight benchmark functions, the results showed the capability of the MBO method significantly outperformed the other five algorithms [21]. In 2020, inspired by a unique mathematical model that slime mould forms the optimal path for connecting food through the positive and negative feedback of the propagation wave, Li et al. proposed the slime mould algorithm (SMA) [22]. In addition, in 2021, by simulating the behavior of African vultures and emperor penguin, respectively, the African vulture optimization algorithm (AVOA) [23] and Aptenodytes Forsteri Optimization (AFO) [24] were designed and provided excellent performance. Similar algorithms are available for moth search algorithm (MSA) [25], colony predation algorithm (CPA) [26], and so on. EA algorithms are inspired by the natural laws of population development and evolution. Among EA algorithms for solving various optimization tasks, the genetic algorithm (GA) [27] and differential evolution algorithm (DE) [28] are undoubtedly the most touted. PhA algorithms rely on physical regulation to suggest solutions to optimization difficulties. Such as multiverse optimizer (MVO) was inspired by the multiverse theory in physics [29]. In addition, the Archimedes optimization algorithm (AOA) is a novel PhA algorithm created with motivations from an exciting regulation of physics Archimedes regulation [30]. In 2021, based on the logic of slope variations computed by the Runge–Kutta method, the Runge–Kutta optimizer (RUN) was proposed and offered outstanding performance on 50 mathematical test functions and four real-world engineering problems [31]. The last set of nature-inspired methods simulates some natural human behaviors. Such as teaching-based learning algorithm (TBLA) [32], socioevolution learning optimization algorithm (SELOA) [33], preaching optimization algorithm (POA) [34], and hunger games search (HGS) [35].

Jellyfish search (JS) optimizer is a high-profile metaheuristic algorithm suggested in 2020, which was roused by the conduct of jellyfish in the ocean [36]. After being compared with ten prominent metaheuristic algorithms on the encyclopedic set of mathematical standard functions and used in a sequence of structural engineering concerns, JS is potentially a flawless algorithm for solving optimization problems. Unavoidably, the original JS algorithm also suffers defects in solving accuracy and premature convergence. Thus, this paper introduces the fractional-order modified strategy, and Gaussian mutation mechanism into the original JS algorithm, jellyfish search algorithm based on fractional-order modified, and Gaussian mutation mechanism (FOGJS). In addition, we apply the improved algorithm to the novel grey model to obtain the optimal order of the forecast model. The contribution of this paper can be outlined as follows:

  An enhanced version of the jellyfish search algorithm with fractional-order modified and Gaussian mutation mechanism is proposed. And the validity of the improved algorithm is discussed on test functions of cec2017 and cec2019 by being compared with the original JS and other ten additional algorithms.
  Based on the fractional time-delayed grey model, we alternate the derivative with a first-order difference. It introduces the trigonometric residual modification technique to design a novel forecast model—a discrete fractional time-delayed grey model with triangular residual correction (TDFTDGM).
  Taking the rural income data of Shaanxi Province as an example, apply the FOGJS to TDFTDGM to search the most suitable fractional order of the forecast model. Then, compared with other optimization algorithms and grey models, the fitting and predicted errors of the FOGJS + TDFTDGM approach are discussed.

The rest of the paper is systematized as tracks. In Section 2, we give the theory of jellyfish search optimizer. The improved JS algorithm is proposed in Section 3.  Section 4 examinations the performance of improved algorithms on miscellaneous test functions.  Section 5 presents the novel grey model and predicts the income of rural residents by different models. Eventually, the work of this paper is abstracted in Section 6.

## 2. The Theory of Jellyfish Search Optimizer

The jellyfish search (JS) is a recent swarm intelligence method founded on jellyfish demeanor in the ocean. The jellyfish's search behavior and movement mode in the ocean encourages the algorithm [36]. As Figure 1 shows, the jellyfish will move with the ocean current or move in the population. Firstly, it is affected by the ocean current. Each jellyfish will follow the ocean current to form a jellyfish gathering. Secondly, once the surrounding food changes, jellyfish will move within the group. These motions are switched by using a time control mechanism.

The different initialization distributions of exact solutions in the search space will affect whether they will eventually fall into local solutions. After observing the typical random methods, it is finally found that the jellyfish search optimizer performs well under the logistic map. The mathematical description is as follows [36]:

(1) $$\begin{array}{c} Z_{i+1}=\alpha Z_{i}\left(1-Z_{i}\right),0\leq Z_{0}\leq 1, \end{array}$$

where *Z*_*i*_ represents the *i-*th jellyfish logistic chaotic value, *Z*_0_ is the first people of developed jellyfish, *Z*_0_ is set between 0 and 1, but *Z*_0_ cannot take some particular values, such as 0.0, 0.25, 0.5, 0.75, 1.0, and *α* is selected to 4.0.

The ocean currents contain a lot of nutrients and are easier to survive, attracting jellyfish. Therefore, the current ocean direction is usually specified by the average vectors from all jellyfish in the ocean group to the jellyfish presently in the optimal situation. The mathematical term of ocean current is as tails [36]:

(2) $$\begin{array}{c} Z_{i}\left(t+1\right)=Z_{i}\left(t\right)+r_{1}\times \left(Z^{*}-\beta \times r_{2}\times \mu \right), \end{array}$$

where *r*_1_ and *r*_2_ are the accidental numerals between 0 and 1, *Z*^*∗*^ is a jellyfish in the most suitable place at present, *β* > 0 is a distribution coefficient, and *β* is usually taken as 3.

The movement in the jellyfish group can be divided into active and passive movements. Initially, when the jellyfish group was just formed, most jellyfish showed passive movement. Passive motion is the movement of jellyfish near its place. At this time, the updated connected place of individual position is

(3) $$\begin{array}{c} Z_{i}\left(t+1\right)=Z_{i}\left(t\right)+\gamma \times r_{3}\times \left(ub-lb\right), \end{array}$$

where *ub* is the upper attached and *lb* is the lower bound of the tracking area, in addition, *γ* is a move coefficient and its value > 0, which is connected to the move length of the jellyfish near its place, and the original algorithm usually takes *γ* = 0.1, and *r*_3_ is an arbitrary number in the range of 0 and 1.

The active movement relies on comparing the food quantity of two jellyfish to judge whether there is relative movement. When the food quantity near the other jellyfish is higher, it will move towards it. The expression of active motion is as tails [36]:

(4) $$\begin{array}{c} Z_{i}\left(t+1\right)=Z_{i}\left(t\right)+r_{4}\times \overset{⟶}{\text{Direction}}, \end{array}$$

where *r*_4_ is a random number between 0 and 1, and $\overset{⟶}{\text{Direction}}$ is used to determine the movement direction of the current jellyfish in the next iteration. This movement always moves in the direction of better food position, and represents the following formula [36]:

(5) $$\begin{array}{c} \overset{⟶}{\text{Direction}}=\left\{\begin{array}{c} Z_{k}\left(t\right)-Z_{i}\left(t\right),\;\text{if }f\left(Z_{i}\right)\geq f\left(Z_{i}\right),\\ Z_{i}\left(t\right)-Z_{k}\left(t\right),\;\text{if }f\left(Z_{i}\right)<f\left(Z_{i}\right), \end{array}\right. \end{array}$$

where *k* is the index of a jellyfish determined haphazardly, and *f* is an objective function.

A time control tool is presented to control the tendency of people between observing the ocean current and driving within the people.  Figure 2 is the allocation of activity within the people. The time control instrument contains a time control function *c*(*t*) and a regular *c*_*o*_, and the time control function is an arbitrary matter that fluctuates from 0 to 1. The term of the time control instrument is as follows [36]:

(6) $$\begin{array}{c} c\left(t\right)=\left(1-\frac{t}{t_{\max}}\right)\times \left(2\times r_{5}-1\right), \end{array}$$

where *t* is the recent iterations, *t*_max_ is the total iterations, and *r*_5_ is a random number between 0 and 1. When *c*(*t*) ≥ *c*_*o*_, swim inward with other passive or active actions; when the randomly generated random number is more significant than (1 − *c* (*t*)), the current people use the inactive motion. Otherwise, the active movement is involved.

## 3. An Improved Jellyfish Search Optimizer

An improved JS algorithm based on fractional-order modified and Gaussian mutation mechanism (FOGJS) is proposed to solve the problem that the jellyfish search algorithm quickly falls into optimal local solution and improves accuracy.

### 3.1. Fractional-Order Modified Strategy

Fractional calculus extends the order of calculus from integer to fraction and recursively deduces the solution limit through the difference approximation of integer calculus, that is, the differentiation and integration with the order of fraction. There are many definitions of derivatives, such as Grünwald–Letnikov, Caputo fractional derivatives [37], Riesz potential [38], and so on. The most commonly used definitions is Grünwald–Letnikov (G-L) [39] definition:

(7) $$\begin{array}{c} {\text{D}}^{\alpha }\left[z\left(t\right)\right]=\underset{T⟶0}{\lim}\left[\frac{1}{T^{\alpha }}\sum_{k=0}^{+\infty }\frac{{\left(-1\right)}^{k}\Gamma \left(\alpha +1\right)z\left(t-kT\right)}{\Gamma \left(k+1\right)\Gamma \left(\alpha -k+1\right)}\right], \end{array}$$

where *α* is the fractional coefficient of a public signal *z*(*t*), Γ is a gamma function, and *T* is the truncation term.

The discrete expression of G-L can be expressed as

(8) $$\begin{array}{c} {\text{D}}^{\alpha }\left[z\left(t\right)\right]=\frac{1}{T^{\alpha }}\sum_{k=0}^{r}\frac{{\left(-1\right)}^{k}\Gamma \left(\alpha +1\right)z\left(t-kT\right)}{\Gamma \left(k+1\right)\Gamma \left(\alpha -k+1\right)}. \end{array}$$

Taking advantage of the fractional learning and training algorithm is easy to leap out of the local extreme points. The jellyfish search algorithm is integrated with the fractional-order modified strategy to adjust the fractional-order by updating the jellyfish position in the ocean current and the jellyfish passive motion position. Let *α* = 4 in equation (8) have the following:

(9) $$\begin{array}{c} {\text{D}}^{\alpha }\left[z\left(t+1\right)\right]\approx z\left(t+1\right)-\alpha z\left(t\right)+\frac{1}{2}\alpha \left(\alpha -1\right)z\left(t-1\right)-\frac{1}{6}\alpha \left(\alpha -1\right)\left(\alpha -2\right)z\left(t-2\right)+\frac{1}{24}\alpha \left(\alpha -1\right)\left(\alpha -2\right)\left(\alpha -3\right)z\left(t-3\right). \end{array}$$

The fractional derivative results are related to the current term and previous state values, and the influence of past events decreases with time. The position update of jellyfish moving under the effect of ocean current and the position update of people passive movement when jellyfish group just formed are equations (2) and (3), respectively.  Figure 3 shows how fractional-order correction affects the update. The left side of equations (2) and (3) is fractional-order G-L, which defines the discrete form when order *α* is 1, and *T* is 1; that is,

(10) $$\begin{array}{c} {\text{D}}^{\alpha }\left[z\left(t+1\right)\right]=r_{1}\times \left(Z^{*}-\beta \times r_{2}\times \mu \right),\\ {\text{D}}^{\alpha }\left[z\left(t+1\right)\right]=\gamma \times r_{3}\times \left(U_{b}-L_{b}\right). \end{array}$$

Therefore, the position update formula of jellyfish affected by ocean current after fractional-order modified is as follows:

(11) $$\begin{array}{c} Z_{i,j}^{t+1}=\alpha Z_{i,j}^{t}-\frac{1}{2}\alpha \left(\alpha -1\right)Z_{i,j}^{t-1}-\frac{1}{6}\alpha \left(\alpha -1\right)\left(\alpha -2\right)Z_{i,j}^{t-2}+\frac{1}{24}\alpha \left(\alpha -1\right)\left(\alpha -2\right)\left(\alpha -3\right)Z_{i,j}^{t-3}+r_{1}\times \left(Z^{*}-\beta \times r_{2}\times \mu \right). \end{array}$$

The update formula of passive motion position of jellyfish after fractional-order modified is

(12) $$\begin{array}{c} Z_{i,j}^{t+1}=\alpha Z_{i,j}^{t}-\frac{1}{2}\alpha \left(\alpha -1\right)Z_{i,j}^{t-1}-\frac{1}{6}\alpha \left(\alpha -1\right)\left(\alpha -2\right)Z_{i,j}^{t-2}+\frac{1}{24}\left(\alpha -1\right)\left(\alpha -2\right)\left(\alpha -3\right)Z_{i,j}^{t-3}+\gamma \times r_{3}\times \left(U_{b}-L_{b}\right). \end{array}$$

It is worth noting that when the terms of 1/120 or 1/720 or higher are multiplied by the remaining terms of equation (8), the values of these terms become negligible and hardly affect the update of position. Therefore, the higher-order terms are discarded.

### 3.2. Gaussian Mutation Mechanism

The Gaussian distribution, also understood as the standard distribution, is a substantial probability distribution in mathematics, artificial intelligence, and other related fields [40]. The Gaussian mutation tool is employed to generate a further variant, which retains a better position by comparing it with the target value of the current optimal individual situation. This mechanism makes the algorithm's local results and global results well balanced [41]. The probability density function (PDF) formula of Gaussian distribution is as tails:

(13) $$\begin{array}{c} G\left(x\right)=\frac{1}{\sqrt{2\pi \sigma }}\exp\left(-\frac{{\left(z-u\right)}^{2}}{2\sigma^{2}}\right), \end{array}$$

where *μ* is the anticipation of Gaussian distribution and *σ* is defined as the standard deviation of Gaussian distribution. We can describe the resulting new mutation location as

(14) $$\begin{array}{c} Z_{i,j}^{new}\left(t+1\right)=Z_{i,j}^{\text{best}}\left(t+1\right)\times \left(1+\theta \times G\left(0,1\right)\right), \end{array}$$

where *θ* is a declining random integer in the range of 0 and 1, *G*(0, 1) is the expected Gaussian distribution, and *Z*_*i*,*j*_^*best*^ is the best location for the current iteration.

### 3.3. Explicit Steps for the Improved Jellyfish Search Optimizer

The fractional-order modified strategy and Gaussian mutation mechanism are presented in JS. The convergence precision of the JS algorithm is effectively enhanced, and the tracking performance of the original JS algorithm is improved. The exact steps of FOGJS are as follows:

**Step 1 .**

Give some parameters associated with FOGJS, such as people dimensions *N*, varying dimension *Dim*, upper set range *ub*, lower set range *lb*, total iterations *M*_*iter*_, the distribution coefficient *β*, and the motion coefficient *γ*.

**Step 2 .**

Aimlessly initialize *N* people size according to chaotic logistic map (equation (1)), and set time *t* = 1.

**Step 3 .**

Compute the fitness value for each people, document the optimal fitness value and the related optimal place *Z*^*∗*^.

**Step 4 .**

While *t* < *M*_*iter*_, compute the control time *c*(*t*) according to equation (6), if *c*(*t*) ≥ 0.5, jellyfish will follow ocean current, update the position of jellyfish by equation (11).

**Step 5 .**

If *c*(*t*) < 0.5, randomly generate an accidental number *r*, ranging from 0 to 1, if *r* > (1 − *c*(*t*)), the jellyfish will update its position by passive motion of equation (12). If *r* ≤ (1 − *c*(*t*)), the position of the jellyfish is computed by active motion according to equation (4).

**Step 6 .**

Judge whether the updated new location crosses the boundary. If yes, the site is set near the border by default. At the same time, the fitness value of individual jellyfish is estimated. If it is more undersized than the optimal value, it is accepted as the new optimal value, and the related position is accepted as the recent optimal position *Z*^*∗*^.

**Step 7 .**

Through the Gaussian mutation mechanism of equation (14), the optimal position is mutated to produce a new solution, and judge its fitness with the optimal solution, to choose whether to update the mutated new solution to the optimal solution.

**Step 8 .**

Update the value of *t* (*t* = *t* + 1), if *t* < *M*_*iter*_, continue Step 4. Otherwise, output the optimal value and the optimal place.

**Step 9 .**

Otherwise, output the optimal value and the optimal place.

To express the enhanced algorithm more obviously, Algorithm 1 gives the pseudocode of the FOGJS. Among them, line 1 is to update the candidate solution position through the logistic chaotic map, lines 9 and lines 14 are the update operation process of applying the fractional modified update formula, and lines 22–26 are the update process after generating the mutation solution through the Gaussian mutation mechanism.  Figure 4 shows the flowchart of the proposed FOGJS algorithm. It can be found that it first defines the parameters listed above and then executes the updated JS based on fractional-order modified. The optimal solution is taken as the initial point of mutation of the Gaussian mutation mechanism. The loop will continue, jump out of the loop when the termination conditions are met and then output the optimal solution of the search.

### 3.4. The Complexity Analysis of FOGJS

The computational complexity of FOGJS mainly relies on three aspects: initialization stage, fitness function evaluation, and coordinated update. The complexity of the initialization stage is O(*N*), where *N* is the number of candidate solutions. Different problems lead to additional complexity of the fitness function, so we will not be concerned about it here. Finally, the complexity update location is O(*N* × *M*), where *M* represents maximum iterations. Therefore, the computational complexity of FOGJS the algorithm is O(*N* × *M*). In the following sections, we will use diverse benchmark functions and actual optimization problems to verify the implementation of FOGJS in dealing with different optimization problems.

## 4. Numerical Examples and Analysis

This part evaluates the comprehensive performance of the improved FOGJS algorithm in solving challenging test functions. Two series of popular functions are used, including 29 cec2017 benchmarks and 10 cec2019 benchmarks [42]. The optimization results of FOGJS are analyzed and compared with other famous optimization algorithms. Meanwhile, to ensure the consistency and reliability of the improved FOGJS, 20 independent tests were conducted on FOGJS and other algorithms. The mean (mean), standard deviation (STD), the worst solution to date, and the best solution to date are reported. To achieve a reasonable comparison, other algorithms considered achieving the same number of iterations 1000 and population 30 as the FOGJS.

### 4.1. Evaluation Index

The following section will analyze the performance differences between the improved FOGJS algorithm and other comparison algorithms through the following evaluation indicators.

#### 4.1.1. The Best Results

(15) $$\begin{array}{c} \text{best}=\text{min}\left({\text{best}}_{1}{\text{,best}}_{2}\text{,}\ldots {\text{,best}}_{\text{runs}}\right), \end{array}$$

where *best*_*i*_ is the best result of each run. *Runs* is the number of runs of each algorithm in each benchmark function, which is taken as 20 in this paper.

#### 4.1.2. The Worst Results

(16) $$\begin{array}{c} \text{worst}=\text{min}\left({\text{worst}}_{1}{\text{,worst}}_{2}\text{,}\ldots {\text{,worst}}_{\text{runs}}\right). \end{array}$$

#### 4.1.3. The Average Value (AVE)

(17) $$\begin{array}{c} \text{Mean}=\frac{1}{\text{Runs}}\sum_{i=1}^{\text{Runs}}{\text{best}}_{i}. \end{array}$$

#### 4.1.4. The Standard Deviation (STD)

(18) $$\begin{array}{c} \text{Std}=\sqrt{\frac{1}{\text{runs}-1}\sum_{i=1}^{\text{runs}}{\left({\text{best}}_{i}-\text{Mean}\right)}^{2}}. \end{array}$$

#### 4.1.5. Wilcoxon's Rank-Sum Test

Wilcoxon's rank-sum test is a nonparametric examination used to test the statistical difference between two sample data sets. Wilcoxon's rank-sum is an effective tool to check whether the FOGJS is significantly better than other comparison algorithms in the general distribution of the examination results.

### 4.2. Parameter Setting

Algorithms with various characteristics are selected to be compared with the FOGJS in this paper. These algorithms include the original JS and other intelligent optimization algorithms, which are differential evolution (DE) [28], multiverse optimizer (MVO) [29], games search (HGS) [35], arithmetic optimization algorithm (AOA) [43], gravity search algorithm (GSA) [44], particle swarm optimization (PSO) [45], whale optimization algorithm (WOA) [46], sparrow search algorithm (SSA) [47], gradient-based optimizer (GBO) [48], lightning search algorithm (LSA) [49], wild horse optimizer (WHOA) [50], crisscross optimization algorithm (CSO) [51], Harris hawks optimization (HHO) [52], atom search optimization (ASO) [53], Aquila optimizer (AO) [19], heap-based optimizer (HBO) [54], seagull optimization algorithm (SOA) [55], grasshopper optimization algorithm (GOA) [56], and lion swarm optimization (LSO) [57]. Considering that the parameters of algorithms will have an impact on performance, these parameters are set the same as those in the corresponding literature, which are shown in Table 1.

### 4.3. Sensitivity Analysis of Parameters

Several JS algorithms introduce parameters that affect the performance when working with improvements, such as the distribution coefficient *β* parameter related to the trend length and the motion coefficient *γ* parameter associated with the update of the position motion length. A sensitivity analysis of the response to parameter changes is now performed to properly understand the effectiveness of these parameters on improving the FOGJS situation.

The coefficient *β* was changed from 0.1 to 1 in steps of 0.1. The coefficient *γ* was changed from 1 to 10 in Step 1. The algorithm was run on 29 cec2017 test functions, where the dimension was set to 30, and the population was set to 30.  Figure 5 shows the average rank obtained for each analysis for the two parameters (*β*, *γ*). The optimal values of the coefficients include for *β* equal to 0.4 and *γ* equal to 2. It is important to note that we set the parameters only when the two strategies of fractional order and Gaussian variation are more effective in improving the JS algorithm. There will be differences with the parameters provided by the JS algorithm. Experiments prove that the FOGJS algorithm is feasible and suitable at *β* = 0.4 and *γ* = 2.

### 4.4. Exploration and Exploitation

The distance between individuals in different dimensions and the overall trend can determine whether the whole tends to be divergence or aggregation. When there is a trend of separation, the difference between each individual in multiple dimensions will become more prominent, which means that each individual explores the space in a differentiated way. This trend will make the algorithm do a more comprehensive exploration of the solution space through the temporary characteristics of the population. In addition, when there is a tendency of aggregation, the population is based on a widely recognized partial exploration space, reducing the differentiation of each individual and doing more detailed exploitation of the region. At the same time, maintaining a good balance between these two modes of exploration and exploitation is a necessary guarantee to find the optimal solution. Usually, algorithms with poorer methods fail to produce satisfactory results.

Studying the trend of convergence plots and the statistical mean, best, worst, and standard deviation over multiple runs do not help us understand an algorithm's exploration process, leading to the failure to solve the speed of accuracy problem faced by an algorithm. Therefore, we resorted to the dimensional diversity measure proposed by Hussain et al. in [58], which calculates the variability between individuals and populations in terms of dimensionality by

(19) $$\begin{array}{c} {\text{Div}}_{k}=\frac{1}{n}\sum_{k=1}^{n}\text{Median}\left(z^{j}\right)-z_{i}^{j},\\ \text{Div}=\frac{1}{\text{Dim}}\sum_{\text{k}=1}^{\text{Dim}}{\text{Div}}_{\text{k}}, \end{array}$$

where *Median*(*z*^*j*^) is the median of *j*th dimension in the whole group, *z*^*j*^_*i*_ is the *j*th dimension of the people *i*, and *n* is the number of the population. After calculating the average Div_*j*_ of each individual, divide the result by Dim to estimate the diversity index of the average dimension.

By obtaining the average diversity of the estimated population after each iteration, we can calculate the exploration and utilization percentage of all iterations according to the following formula:

(20) $$\begin{array}{c} \text{Exploration}\%=\frac{\text{Div}}{{\text{Div}}_{\text{max}}}\times 100,\\ \text{Exploitation}\%=\frac{\left|{\text{Div}-\text{Div}}_{\text{max}}\right|}{{\text{Div}}_{\text{max}}}\times 100, \end{array}$$

where Div is the average diversity of the population in each iteration and *Div*_*max*_ is the maximum of the average variety in all iterations. *Exploration*% and *Exploitation*% are the exploration and development percentages of iterations, respectively.

Figure 6 shows the exploration and exploitation diagrams of FOGJS for some of the cec2017 test functions (cec03, cec06, cec09, cec10, cec11, cec12, cec13, cec14, cec16, cec17, cec19, cec20, cec22, cec24, and cec27). From cec03, cec11, cec20, and cec24, we can find that FOGJS has a high exploration rate at the beginning of the iteration and a rapid transition to a high exploitation rate in the middle and finally finishes the iteration with a high exploitation profile. This process indicates that the higher exploration rate in the early stage of FOGJS ensures the global search and prevents getting into the optimal local solution, while the higher exploitation rate in the later stage ensures the higher accuracy of the optimal solution. And in cec10, cec14, cec17, and cec20 test functions, the exploration and exploitation maintain almost the same ratio throughout the iterations, indicating that FOGJS can ensure the balance between the two when handling these test functions. Whereas in cec06, cec09, cec12, cec13, and cec19, the exploitation rate has been dominant throughout the iterative process, and in cec27, the opposite is true.

In summary, FOGJS has different strategies in dealing with varying test functions and therefore has a solid dynamic and adaptable nature.  Figure 7 shows the histogram of the percentage of both exploration and exploitation for different test functions. As can be seen, there are 12 test functions with more than 50% exploitation, while at cec10, cec20, and cec27 while more focused on exploration.

### 4.5. Comparison Results Using cec2017 Test Functions

To further prove the performance of the improved JS algorithm, a challenging set of test functions named cec2017 is selected to be solved. It contains 29 functions, at least half of which are challenging mixed and combined functions. To evaluate the stability of the improved FOGJS performance, these functions are used to test FOGJS. Meanwhile, the FOGJS has achieved 1000 iterations and 30 population sizes for 20 independent operations. The results are compared with other excellent algorithms, including JS [36], GSA [44], MVO [29], WOA [46], GOA [56], LSO [57], HHO [52], ASO [53], AOA [43], and AO [19]. The AVE (average value) and STD (standard deviation) values of the benchmark test bench considered are calculated through the executed algorithm. In addition, to make the data more convincing, the last few rows of the table contain the statistical results of the Wilcoxon rank-sum test, where “+” indicates that the results of other algorithms are better than FOGJS, “−” means the opposite, and “=” suggests that there is no significant contrast between FOGJS and different comparison methods. The best average obtained by 12 algorithms in tables is also drawn in bold.

Table 2 provides the evaluation results of the best solution to date. The average rank of the FOGJS is 2.28, ranking first. Among them, the FOGJS provides the best results of all algorithms in 10 functions and also shows strong competitiveness in other functions. For other algorithms, MVO ranks second, second only to FOGJS, and has successfully implemented 10 functions, but it has poor competitiveness in other functions. JS and CSO successfully implemented 6 and 3 functions, respectively, while GSA, WOA, GOA, LSO, HHO, ASO, AOA, and AO did not show the best performance. In conclusion, the FOGJS is superior to other optimization algorithms in accuracy and occupies the first place. In addition, the ranking of the original JS is 2.69, which is lower than that of the FOGJS. It can be seen that the fractional-order modified strategy and Gaussian mutation mechanism improve the effective exploration ability of the JS in finding the optimal solution. The FOGJS algorithm can search for better solutions with faster convergence rates established on the actual algorithm. The results of the Wilcoxon rank-sum test are shown in the final row of Table 2. The Wilcoxon rank-sum test results of JS, GSA, CSO, MVO, WOA, and GOA are 3/26/0, 1/4/24, 2/12/15, 9/10/10, 0/2/27, 1/5/23, LSO, HHO, ASO, AOA, and AO are 0/0/29, 1/2/26, 0/2/27, 0/1/28, and 1/4/24, respectively.  Figure 8 displays the average convergence process of 29 test functions in 30-dimensions. By analyzing the curve, it can be found that the iterative curve of FOGJS can escape the local solution and connect to the approximate optimal solution in the early phase of iteration, and the optimization will be found near the optimal solution in the later development stage. Specifically, in the 30-dimensional convergence curve, the FOGJS shows that the convergence effects of cec01, cec05, cec16, cec21, and cec29 are more obvious. This observation shows that the FOGJS can be regarded as one of the most reliable algorithms.  Figure 9 shows the box plots of different algorithms. Obviously, in most test functions, the box of the FOGJS algorithm is more concentrated, and its target distribution is smaller than other improved algorithms, which shows that the enhanced algorithm has good stability. The results of the Wilcoxon rank-sum test are shown in Table 3.  Table 4 shows the number of function evaluations and execution times for each comparison algorithm. It can be found that FOGJS has a longer execution time compared to the original algorithm, which is due to the added improvement strategy. FOGJS has a shorter execution time than the GOA and ASO algorithm but still requires a long running time. NFFEs are the number of equation evaluations of an algorithm, which is another expression of the execution efficiency of an algorithm. JS, GSA, MVO, WOA, ASO, and AOA all have smaller NFFEs, while FOGJS has 60030 NFFEs in one run.

### 4.6. Comparison Results Using cec2019 Test Functions

This section describes in detail the analysis of FOGJS results when tested with the ten functions of the latest CEC benchmark (cec2019). All results are obtained after 20 independently runs by set the population size as 30 and the iterations as 1000 times. The results were compared with JS [36], PSO [45], DE [28], LSA [49], GBO [48], SOA [55], HGS [35], SSA [47], HBO [54], WHOA [50], and AOA [43]. As shown in Table 5, in the whole process of the function, the worst value, average value, the best value, and the STD value are compared through the considered algorithm. In addition, the results of the Wilcoxon rank-sum test are shown in Table 6. According to the data results in Table 5, the average rank of the FOGJS is 2.8, ranking first. FOGJS provides the best results in cec01, cec02, cec08, and cec10. Compared with other algorithms, FOGJS is also very competitive in other test functions. WHOA ranks second, ranking worse than FOGJS. At the same time, it successfully implements one function and shows good competitiveness in other functions. For other comparison functions, HBO successfully implemented four functions, while SSA and HGS successfully implemented one function. The results show that the improved FOGJS has better convergence accuracy and accuracy than other algorithms. The last row of Table 5 gives the average and rank ranking. The Wilcoxon rank-sum test results of JS, PSO, DE, GBO, LSA, and SOA algorithms are 1/5/4, 0/2/8, 0/0/10, 2/3/5, 1/4/5, and 0/0/10, respectively. The Wilcoxon rank-sum test results of SSA, HGS, HBO, WHOA, and AOA are 0/5/5, 0/6/4, 4/2/4, 1/5/4, and 0/0/10, respectively.  Figure 10 shows the convergence curve of 10 test functions. FOGJS can get closer to the optimal solution faster than other algorithms by analyzing the curve. At the same time, it will find the optimization near the optimal solution in the middle development stage of iteration and replace the original solution with the newly found better solution. Specifically, FOGJS shows that the convergence effects of cec01, cec02, cec04, cec06, and cec08 are apparent in the convergence curve.  Figure 11 shows the box plot of 12 algorithms in 10 test functions. We can find that the length of the FOGJS box is small, and there are few outliers when combining the results of 20 runs, thus showing the stability and balance of FOGJS.  Table 7 shows the number of function evaluations and execution times for each comparison algorithm.

## 5. Income Forecast Model of Rural Resident Based on Improved Jellyfish Search Optimizer

Agriculture, rural areas, and farmers are important issues for the long-term stability of the country. In order to adopt a series of corresponding policies to benefit and support agriculture, the forecast of farmers' income trend becomes the task need to be solve. Disposable income represents the sum of the ultimate consumer spending and savings obtained by residents, which can play an important role in estimating per capita consumption power and understanding the productivity of an area. Thus, this paper discusses the per capita disposable income of rural residents in Shaanxi Province. For ease to be understood, per capita disposable income of rural resident in this paper is simply referred to as income of rural resident. As Figure 12 shows, income of rural resident in Shaanxi Province is increasing from 1989 to 2020. In this section, a novel discrete fractional time-delayed grey model is established to solve the problem of income forecast.

### 5.1. Income Forecast Model Based on Improved Jellyfish Search Optimizer

#### 5.1.1. Establishment of the TDFTDGM Model

Grey model (GM) is a popular predicted approach by establishing a grey differential prediction model through a small amount of incomplete information and the development trend of the internal system is described, which has been widely applied to population forecast, economy forecast, and climate prediction. In [16], a fractional time-delayed grey model was proposed. However, the conversion from the discrete equation to the continuous equation will bring conversion error, which will decrease the accuracy of prediction. Thus, this paper establishes a novel discrete fractional time-delayed grey model with triangular residual correction (TDFTDGM).

Firstly, given a raw nonnegative data set *Z*^(0)^=(*z*^(0)^(1), *z*^(0)^(2), ⋯, *z*^(0)^(*n*)). Then, calculate the *m*-order accumulated sequence *Z*^(*m*)^=(*z*^(*m*)^(1), *z*^(*m*)^(2), ⋯, *z*^(*m*)^(*n*)) by

(21) $$\begin{array}{c} z^{\left(m\right)}\left(k\right)=\sum_{i=1}^{k}\left(\begin{array}{c} k-i+m-1\\ k-i \end{array}\right)z^{\left(0\right)}\left(i\right),k=1,2,\cdots ,n, \end{array}$$

where $\left(\begin{array}{c} k-i+m-1\\ k-i \end{array}\right)=\left(k-i+m-1\right)\left(k-i+m-2\right)\cdots \left(m+1\right)m/\left(k-i\right)!$.

Differential equation (23) is the basic fractional grey model (FGM) with order *m*:

(22) $$\begin{array}{c} \frac{\text{d}z^{\left(m\right)}\left(t\right)}{\text{d}t}+az^{\left(m\right)}\left(t\right)=bt^{\left(m\right)}+c. \end{array}$$

For the derivative of the left of equation (22), the first backward difference can be approximately expressed by equation (23) when *t* = *k*:

(23) $$\begin{array}{c} {\left(\frac{\text{d}z^{\left(m\right)}\left(t\right)}{\text{d}t}\right)}_{t=k}\approx \underset{\Delta t⟶1}{\lim}\frac{z^{\left(m\right)}\left(k\right)-z^{\left(m\right)}\left(k-\Delta t\right)}{\Delta t}\\ =z^{\left(m\right)}\left(k\right)-z^{\left(m\right)}\left(k-1\right). \end{array}$$

Thus, when *t* = *k*, the left of (22) can be approximated by follows:

(24) $$\begin{array}{c} {\left(\frac{\text{d}z^{\left(m\right)}\left(t\right)}{\text{d}t}+az^{\left(m\right)}\left(t\right)\right)}_{t=k}\approx z^{\left(m\right)}\left(k\right)-z^{\left(m\right)}\left(k-1\right)+az^{\left(m\right)}\left(k\right)\\ ={\left(1+az\right)}^{\left(m\right)}\left(k\right)-z^{\left(m\right)}\left(k-1\right). \end{array}$$

Substituting equations (24) into (22), equation (25) can be obtained:

(25) $$\begin{array}{c} \left(1+a\right)z^{\left(m\right)}\left(k\right)-z^{\left(m\right)}\left(k-1\right)=bk^{\left(m\right)}+c, \end{array}$$

where $k^{\left(m\right)}=\sum_{i=1}^{k}\left(\begin{array}{c} k-i+m-1\\ k-i \end{array}\right)\cdot i$ is the time delay term with *m*-order.

Then, discrete formula (25) can be obtained by letting *β*_1_=1/1+*a*, *β*_2_=*b*/1+*a*, *β*_3_=*c*/1+*a*:

(26) $$\begin{array}{c} z^{\left(m\right)}\left(k\right)=\beta_{1}z^{\left(m\right)}\left(k-1\right)+\beta_{2}k^{\left(m\right)}+\beta_{3}. \end{array}$$

Equation (26) is the discrete fractional time-delayed grey model (FTDGM), which can be expressed by matrix:

(27) $$\begin{array}{c} B\beta =Y, \end{array}$$

where $B=\left[\begin{array}{ccc} z^{\left(m\right)}\left(1\right) & 2^{\left(m\right)} & 1\\ z^{\left(m\right)}\left(2\right) & 3^{\left(m\right)} & 1\\ \vdots & \vdots & \vdots \\ z^{\left(m\right)}\left(n-1\right) & n^{\left(m\right)} & 1 \end{array}\right],Y=\left[\begin{array}{c} z^{\left(m\right)}\left(2\right)\\ z^{\left(m\right)}\left(3\right)\\ \vdots \\ z^{\left(m\right)}\left(n\right) \end{array}\right],\beta =\left[\begin{array}{c} \beta_{1}\\ \beta_{2}\\ \beta_{3} \end{array}\right]$.

If the fractional order *m* was determined, parameters *β*1, *β*2, and *β*3 can be estimated by the least squares solution as equation (28):

(28) $$\begin{array}{c} \hat{\beta }={\left[{\hat{\beta }}_{1},{\hat{\beta }}_{2},{\hat{\beta }}_{3}\right]}^{Τ}={\left(B^{Τ}B\right)}^{-1}B^{Τ}Y. \end{array}$$

Then, the value of ${\hat{z}}^{\left(r\right)}\left(k\right)$ can be obtained by equation (29) after determining the parameters *β*1, *β*2, and *β*3:

(29) $$\begin{array}{c} {\hat{z}}^{\left(m\right)}\left(k\right)={\hat{\beta }}_{1}z^{\left(m\right)}\left(k-1\right)+{\hat{\beta }}_{2}k^{\left(m\right)}+{\hat{\beta }}_{3}\\ =z^{\left(0\right)}\left(1\right)\cdot {\left({\ddot{\beta }}_{1}\right)}^{\left(k-1\right)}+\sum_{i=2}^{k}\left({\hat{\beta }}_{2}i^{\left(m\right)}+{\hat{\beta }}_{3}\right)\cdot {\left({\hat{\beta }}_{1}\right)}^{\left(k-i\right)}. \end{array}$$

Finally, the predicted value ${\hat{Z}}^{\left(0\right)}=\left({\hat{z}}^{\left(0\right)}\left(1\right),{\hat{z}}^{\left(0\right)}\left(2\right),\cdots ,{\hat{z}}^{\left(0\right)}\left(n\right)\right)$ is obtained by *m*-order inverse fractional-order accumulation:

(30) $$\begin{array}{c} {\hat{z}}^{\left(0\right)}\left(k\right)={\left({\hat{z}}^{\left(m\right)}\left(k\right)\right)}^{\left(-m\right)}=\sum_{i=1}^{k}\left(\begin{array}{c} k-i-m-1\\ k-i \end{array}\right){\hat{z}}^{\left(m\right)}\left(i\right). \end{array}$$

Furthermore, the prediction precision of the model can be improved by analyzing the error between the raw data and predicted data. Thus, this paper introduces the triangular residual correction function into the discrete fractional time-delayed grey model to obtain a new prediction model with higher precision. According to the predicted value in equation (30), the residual error sequence can be calculated as follows:

(31) $$\begin{array}{c} r\left(k\right)=z^{\left(0\right)}\left(k\right)-{\hat{z}}^{\left(0\right)}\left(k\right),k=2,3,\cdots ,n. \end{array}$$

In addition, the definition of the triangle model is shown as

(32) $$\begin{array}{c} r\left(k+1\right)=b_{0}+b_{1}k+b_{3}\sin\frac{2\pi k}{T}+b_{4}\cos\frac{2\pi k}{T}+\varepsilon_{k+1},k=1,3,\cdots ,n-1, \end{array}$$

where *ɛ* is the random error and *T* is the parameter of time period. *b*_1_, *b*_2_, *b*_3_, and *b*_4_ are obtained by the least squares solution as

(33) $$\begin{array}{c} b={\left[b_{0},b_{1},b_{2},b_{3}\right]}^{Τ}={\left(C^{Τ}C\right)}^{-1}C^{Τ}R, \end{array}$$

where $C=\left[\begin{array}{cccc} 1 & 1 & \sin2\pi /T & \cos2\pi /T\\ 1 & 2 & \sin4\pi /T & \cos4\pi /T\\ \vdots & \vdots & \vdots & \vdots \\ 1 & n-1 & \sin2\left(n-1\right)\pi /T & \cos2\left(n-1\right)\pi /T \end{array}\right],R=\left[r\left(2\right),r\left(3\right)\cdots ,r\left(n\right)\right]$.

Submitting *b*_1_, *b*_2_, *b*_3_, and *b*_4_ into (32), the finial predicted values *Z*^*∗*^=(*z*^*∗*^(1), *z*^*∗*^(2), ⋯, *z*^*∗*^(*n*)) can be obtained as follows:

(34) $$\begin{array}{c} \left\{\begin{array}{c} z^{*}\left(1\right)=z^{\left(0\right)}\left(1\right),\\ z^{*}\left(k\right)={\hat{z}}^{\left(0\right)}\left(k\right)+\hat{r}\left(k\right),k=2,3,\ldots , \end{array}\right. \end{array}$$

when *k* ≤ *n*, ${\hat{z}}^{\left(0\right)}\left(k\right)$ are the fitting values of the raw data. And when *k* > *n*, ${\hat{z}}^{\left(0\right)}\left(k\right)$ are the predicted values.

#### 5.1.2. Optimization Model Based on the FOGJS Algorithm

Obviously, once given the order *m*, the predicted value can be calculated by the above TDFTDGM model. Regarding the order *m* as a variable, the improved jellyfish search optimizer just can be employed to search the most suitable *m* to obtain predicted value with higher precision. Thus, an optimization model can be established by minimizing the mean absolute percentage error between the calculated values and the actual value. The final established optimization model is shown as equation (35).

The data set used in this experiment is the income of rural residents from 1989 to 2020 in Shaanxi Province. The data from 1989 to 2013 are used as training data, and the rest is regarded as test data. Then, the process for FOGJS to solve the rural resident's income forecasting model is displayed in Figure 13:

(35) $$\begin{array}{c} \min\arg\left(f\left(m\right)\right)=\frac{1}{n-1}\sum_{k=2}^{n}\left|\frac{z^{*}\left(k\right)-z^{\left(0\right)}\left(k\right)}{z^{\left(0\right)}\left(k\right)}\right|\times 100\%,\\ s.t.\left\{\begin{array}{c} {\left[{\hat{\beta }}_{1},{\hat{\beta }}_{2},{\hat{\beta }}_{3}\right]}^{Τ}={\left(B^{Τ}B\right)}^{-1}B^{Τ}Y\\ {\hat{z}}^{\left(m\right)}=\left(k\right)z^{\left(m\right)}\left(1\right)\cdot {\left({\hat{\beta }}_{1}\right)}^{\left(k-1\right)}+\sum_{i=2}^{k}\left({\hat{\beta }}_{2}|i^{\left(r\right)}|+|{\hat{\beta }}_{3}\right)\cdot {\left({\hat{\beta }}_{1}\right)}^{\left(k-i\right)},\\ {\left[b_{0},b_{1},b_{2},b_{3}\right]}^{Τ}={\left(C^{Τ}|C\right)}^{-1}C^{Τ}R\\ \hat{r}\left(k+1\right)=b_{0}+b_{1}k+b_{3}\sin\frac{2\pi k}{T}+b_{4}\cos\frac{2\pi k}{T}+\varepsilon_{k+1},k=1,3,\ldots ,n-1,\\ z^{*}\left(1\right)=z^{\left(0\right)}\left(1\right),\\ z^{*}\left(k\right)={\hat{z}}^{\left(0\right)}\left(k\right)+\hat{r}\left(k\right),k=2,3,\ldots , \end{array}\right. \end{array}$$

### 5.2. The Comparison Results Based on Different Optimization Algorithms

In Section 5.1, an optimization model for resident income forecasting is proposed by considering the order *m* as a decision variable. However, lots of optimization algorithms can be used to solve the optimization model. Thus, to verify the validity of the prediction model based on the FOGJS algorithm, the original JS algorithm and other algorithms are employed to solve this optimization model. The selected comparison algorithms are the original JS algorithm [36], Aquila optimizer (AO) [19], sine cosine algorithm (SCA) [59], grey wolf optimizer (GWO) [60], rat swarm optimizer (RSO) [61], seagull optimization algorithm (SOA) [55], DE [28], and PSO algorithm [45]. Meanwhile, to reflect the efficiency of the algorithm, the number of iterations is set as 30 times to highlight the ability of the algorithm to solve problems in a short time. Here, the parameters of the FOGJS algorithm are the same as the results obtained by the sensitivity analysis in Section 4.3. That is, *β* = 0.4 and *γ* = 2. All algorithms run 10 times independently setting the size of the population as 50. Then, Table 8 provides the results after 10 times runs, including the best value (Best), the average value (Mean), the worst value (Worst), and the standard deviation (Std). According to the error between predicted data and the real data in Table 8, the FOGJS algorithm is the most suitable one to solve the predicted model than others, because it has the best performance on all measure indexes. Though JS, DE GWO, and PSO also perform well on the best values, they are much worse than the FOGJS algorithm in terms of average values. It illustrates other algorithms are highly susceptible to local optimums, thus causing instability of the solutions.

Figure 14 also supports the above conclusion through boxplots. The lowest position and the smallest height of the box plotted by the obtained results indicate that the FOGJS algorithm has strong robustness in solving the problem. Both JS and DE algorithms have some outliers, showing that the quality of the solutions is easily affected by other factors, which needs to be avoided in practice applications. Moreover, Figure 15 shows the convergence curves of different algorithms in solving the predicted model of resident income. The FOGJS algorithm has the fastest convergence speed in the early period of iteration, especially being compared with the original JS algorithm. That is, the fractional-order modified mechanism improves the quality of the whole population, speeding up the convergence rate to the optimal solution. In the later stages of the search, Gaussian mutation also plays a role in avoiding local optimums, which can be observed in the enlarged subplot.

### 5.3. The Comparison Results of Different Predicted Models

According to the analysis of Section 5.2, the predicted model based on FOGJS algorithm is effective in solving the predicted problem of resident income. Then, the TDFTDGM + FOGJS approach also needs to be compared with other classical predicted models. In this section, the other six predicted approaches are selected, including GM [12], DGM [14], TRGM [13], FANGBM [15], FTDGM [16], and DFTDGM.  Table 9 displays the measure indicators in the prediction of resident income to illustrate the difference of all models. To compare different models more fairly, two types of errors will be calculated. The fitting error is the error between data obtained by models and training data. And the predicted error represents the error between data obtained by models and test data.

Table 10 displays the fitting results obtained by different forecast models. In addition, Table 11 shows the fitting error compared with the actual data. Obviously, the TDFTDGM predicted model shows better performance than others on two evaluation indicators, which is marked in bold. Compared with GM, TRGM has a smaller fitting error. Meanwhile, under similar results in MAPE and RMSPE, TDFTDGM performs significantly better than DFTDGM on MAE and MSE, which illustrates that applying the triangular residual correction method into the original model is an effective method to improve prediction accuracy.

Figure 16 shows the fitting curve of different models. The FTDGM and FANGBM models perform well before about 2004. However, after that, the fitting data of FTDGM and FANGBM differ greatly from the real income data. That is, these two models have great defects when facing a set of data with large fluctuation. After discretizing the FTDGM model, DFTDGM overcomes this disadvantage as shown in the yellow curve in Figure 16. However, after 2010, the gap between the income data obtained using the DFTDGM model and the real income become larger. The red curve of the TDFTDGM model is closer to the real data for all fitting data with time growth, which means the trigonometric correction function further improves the accuracy of the prediction model to let it more suitable for long-term forecasting. The analysis of the combined results shows that the fitted data obtained by TDFTDGM model are more in line with the actual income changes in the process.

Table 12 shows the predicted results obtained by all models, and the predicted error is summarized in Table 13. For the predicted error, the advantages of TDFTDGM are even more obvious on all four evaluation indexes. In addition, the predicted error of the FANGBM model is large, though it provides great performance in fitting results. The mean absolute percentage error (MAPE) and root mean square percentage error (RMSPE) of FANGBM are all over 10, which means its poor prediction ability.

Meanwhile, it can be observed in Figure 17 that the predicted curve of TRGM is moving away from the real curve with the increase of years. Thus, though the TRGM model also has smaller MAPE and RMSPE, the predicted precision will decrease if the predicted data after 2020 is still needed. However, the predicted data obtained by the TDFTDGM model is able to maintain fluctuations in the vicinity of the real data. Hence, the proposed model with triangular residual correction is superior to others and can provide more reliable and informative predictions.

The income of rural residents in the next five years (2021–2025) is also predicted and shown in Table 14. In addition, Figure 18 is plotted by the predicted data. The curves of TRGM and FTDGM are growing too fast and slow, respectively, which are not conform to the trend of income growth. The red curve's growth rate of the TDFTDGM model is more stable, which is more suitable for the long-term forecast of rural residents' income. Moreover, due to the different performance on fitting and predicted error, Figure 19 draws the bar graphs to discuss the comprehensive performance of different models. On the four-measure indexes, the proposed TDFTDGM model has outstanding advantages over other models. That is, by introducing the trigonometric correction function and FOGJS into the discrete fractional time-delayed grey model, it becomes a competitive forecasting method in practical application.

## 6. Conclusion and Future Work

This paper predicts the rural resident income by combing the TDFTDGM model and FOGJS algorithm. Firstly, the fractional-order modified and Gaussian mutation mechanisms are introduced into the original JS algorithm. After analyzing the effect of different parameters, more suitable parameters are selected in the FOGJS algorithm to improve its capacity. Then, from the exploration and exploitation diagrams, the FOGJS algorithm keeps a balance between the two capacities. Meanwhile, by being compared with different kinds of algorithms on classical test functions, the FOGJS algorithm offers outstanding performance. For the solution precision, the improved algorithm ranks first in terms of mean rank on both cec2017 and cec2019. From the convergence curves and box plots, it can be observed that the FOGJS algorithm has advantages of convergence speed and stability. Moreover, the results of the Wilcoxon rank-sum test further support the conclusion that the introduction of improvement strategies forms the special search mechanism to provide superior performance.

Secondly, the discrete fractional time-delayed grey model with triangular residual correction is established. In addition, the FOGJS algorithm is used to optimize the order of the model. The experiment of income forecasting is divided into two parts. On the one hand, the original JS algorithm and the other seven popular algorithms are selected to solve the TDFTDGM model to be compared with the FOGJS algorithm. Results show that FOGJS algorithm has outstanding performance on precision and convergence speed, which indicates that the FOGJS + TDFTDGM approach is an effective tool for prediction of resident income. On the other hand, the FOGJS + TDFTDGM approach is compared with other six prediction models. Experiments show that TDFTDGM model obtains the predicted data closer to the real income data. Thus, a conclusion can be deduced that TDFTDGM model is more suitable for the long-term prediction of volatile data. The combination between TDFTDGM and FOGJS algorithm also provides an idea to determine the parameters in the forecast model.

In future work, the fractional-order modified and Gaussian mutation mechanism may also be suitable choices for some metaheuristic algorithms (e.g., MRFO algorithm [62] and hybrid arithmetic optimization algorithm [63]) to improve their performance. Moreover, the TDFTDGM model can deal with forecast problems in other fields, such as population forecast, climate forecast, and resource forecast.

## Figures and Tables

**Figure 1:** The simulation of ocean current and swarm.

**Figure 2:** The direction of movement of jellyfish.

**Figure 3:** FOC memory property-based *Z* concept.

**Figure 4:** Flowchart for the proposed FOGJS optimization algorithm.

**Figure 5:** The average rank of FOGJS algorithms with different parameters on cec2017.

**Figure 6:** The exploration and exploitation diagrams of FOGJS. (a). cec03. (b) cec06. (c) cec09. (d) cec10. (e) cec11. (f) cec12. (g) cec13. (h) cec14. (i) cec16. (j) cec17. (k) cec19. (l) cec20. (m) cec22. (n) cec24. (o) cec27.

**Figure 7:** The histogram of the percentage of both exploration and exploitation.

**Figure 8:** The convergence curves of the FOGJS and other comparison algorithms on cec2017 functions. (a) cec01. (b) cec03. (c) cec04. (d) cec05. (e) cec06. (f) cec06. (g) cec08. (h) cec09. (i) cec10. (j) cec11. (k) cec12. (l) cec13. (m) cec14. (n) cec15. (o) cec16. (p) cec17. (q) cec18. (r) cec19. (s) cec20. (t) cec21. (u) cec22. (v) cec23. (w) cec24. (x) cec25. (y) cec26. (z) cec27. (z.1) cec28. (z.2) cec29. (z.3) cec30.

**Figure 9:** Box plot of the FOGJS algorithm and other algorithms on cec2017 functions (red minus ⟶ median; red plus ⟶ outlier). (a) Boxplot of cec01. (b) Boxplot of cec03. (c) Boxplot of cec04. (d) Boxplot of cec05. (e) Boxplot of cec06. (f) Boxplot of cec07. (g) Boxplot of cec08. (h) Boxplot of cec09. (i) Boxplot of cec10. (j) Boxplot of cec11. (k) Boxplot of cec12. (l) Boxplot of cec13. (m) Boxplot of cec14. (n) Boxplot of cec15. (o) Boxplot of cec16. (p) Boxplot of cec17. (q) Boxplot of cec18. (r) Boxplot of cec19. (s) Boxplot of cec20. (t) Boxplot of cec21. (u) Boxplot of cec22. (v) Boxplot of cec23. (w) Boxplot of cec24. (x) Boxplot of cec25. (y) Boxplot of cec26. (z) Boxplot of cec27. (z.1) Boxplot of cec28. (z.2) Boxplot of cec29. (z.3) Boxplot of ce30.

**Figure 10:** The convergence curves of the FOGJS and other intelligent algorithms on cec2019 test functions. (a) cec01. (b) cec02. (c) cec03. (d) cec04. (e) cec05. (f) cec06. (g) cec07. (h) cec08. (i) cec09. (j) cec10.

**Figure 11:** Box plot of the FOGJS and other algorithms for cec2019 test functions (red minus ⟶ median; red plus⟶ outlier). (a) Boxplot of cec01. (b) Boxplot of cec02. (c) Boxplot of cec03. (d) Boxplot of cec04. (e) Boxplot of cec05. (f) Boxplot of cec06. (g) Boxplot of cec07. (h) Boxplot of cec08. (i) Boxplot of cec09. (j) Boxplot of cec10.

**Figure 12:** Income of rural resident from 1989 to 2020 in Shaanxi Province.

**Figure 13:** The process of the TDFTDGM prediction model based on the FOGJS algorithm.

**Figure 14:** The boxplots of different algorithms.

**Figure 15:** The convergence curves of different algorithms.

**Figure 16:** Fitting curves of income by different forecast models.

**Figure 17:** Predicted curves of income by different forecast models.

**Figure 18:** The curves of resident income from 2021 to 2025 through various forecast models.

**Figure 19:** Comprehensive comparison of different forecast models. (a) MAE. (b) MAPE. (c) MSE. (d) RMSPE.

**Algorithm 1:** The proposed FOGJS.

**Table 1:** Parameters setting.

Algorithm	Parameters	Values
AOA [43]	Control parameter	*µ* = 0.499
	Sensitive parameter	*a* = 5
GSA [44]	ElitistCheck, Rpower, Rnorm, alpha, *G*0	1, 1, 2, 20, 100
PSO [45]	c_1_, c_2_, v_Max_, w	2, 2, 6, 1
WOA [46]	A	Decreased from 2 to 0
	b	2
SSA [47]	Leader position update probability	*c*3 = 0.5
GBO [48]	*β*_min_, *β*_min_	0.2, 1.2
	*pr*	0.5
SOA [48]	Control parameter (A)	[2, 0]
	*fc*	2
JS [36]	*β*	3
	*γ*	0.1
LSA [49]	Channel time	10
DE [28]	Scalingfactor, crossoverprobability	0.5, 0.5
WHO [50]	Crossover percentage	PC = 0.13
	Stallions percentage (number of groups)	PS = 0.2
	Crossover	Mean
MVO [29]	WEP_Max, WEP_Min	1, 0.2

**Table 2:** Results of FOGJS and different comparison methods on cec2017 test functions.

Function	Index	Algorithms											
		JS	GSA	CSO	MVO	WOA	GOA	LSO	HHO	ASO	AOA	AO	FOGJS
cec01	AVE	1.68*E* + 06	3.17*E* + 07	2.13*E* + 08	5.40*E* + 05	1.61*E* + 09	4.82*E* + 08	5.55*E* + 10	2.99*E* + 07	4.93*E* + 10	7.16*E* + 10	6.19*E* + 08	5.80*E* + 05
	STD	2.65*E* + 06	6.36*E* + 07	7.85*E* + 07	2.29*E* + 05	7.47*E* + 08	6.91*E* + 08	9.22*E* + 09	6.42*E* + 06	2.29*E* + 10	7.95*E* + 09	2.82*E* + 08	1.30*E* + 06
	Rank	3	5	6	1	9	7	11	4	10	12	8	2

cec03	AVE	4.74*E* + 04	9.74*E* + 04	8.87*E* + 04	1.68*E* + 03	2.73*E* + 05	6.38*E* + 04	8.47*E* + 04	4.07*E* + 04	3.66*E* + 05	9.19*E* + 04	5.46*E* + 04	3.79*E* + 04
	STD	8.78*E* + 03	1.20*E* + 04	2.72*E* + 04	8.95*E* + 02	6.69*E* + 04	3.38*E* + 04	8.51*E* + 03	6.32*E* + 03	1.17*E* + 05	3.13*E* + 03	8.44*E* + 03	5.46*E* + 03
	Rank	4	10	8	1	11	6	7	3	12	9	5	2

cec04	AVE	5.39*E* + 02	6.62*E* + 02	6.01*E* + 02	4.97*E* + 02	8.48*E* + 02	5.60*E* + 02	1.61*E* + 04	5.60*E* + 02	1.23*E* + 04	2.54*E* + 04	6.57*E* + 02	5.39*E* + 02
	STD	2.60*E* + 01	1.02*E* + 02	8.15*E* + 01	1.37*E* + 01	1.56*E* + 02	9.31*E* + 01	4.27*E* + 03	4.31*E* + 01	7.78*E* + 03	4.93*E* + 03	6.68*E* + 01	2.81*E* + 01
	Rank	2	8	6	1	9	5	11	4	10	12	7	3

cec05	AVE	6.58*E* + 02	7.42*E* + 02	6.78*E* + 02	6.18*E* + 02	8.22*E* + 02	8.28*E* + 02	9.02*E* + 02	7.51*E* + 02	8.14*E* + 02	9.21*E* + 02	7.03*E* + 02	6.71*E* + 02
	STD	2.93*E* + 01	2.76*E* + 01	3.30*E* + 01	4.56*E* + 01	4.56*E* + 01	7.64*E* + 01	3.48*E* + 01	4.05*E* + 01	1.03*E* + 02	2.24*E* + 01	3.33*E* + 01	6.16*E* + 01
	Rank	2	6	4	1	9	10	11	7	8	12	5	3

cec06	AVE	6.23*E* + 02	6.58*E* + 02	6.01*E* + 02	6.32*E* + 02	6.76*E* + 02	6.77*E* + 02	6.82*E* + 02	6.66*E* + 02	6.62*E* + 02	6.67*E* + 02	6.55*E* + 02	6.27*E* + 02
	STD	7.21*E* + 00	3.61*E* + 00	1.09*E* + 00	1.48*E* + 01	1.13*E* + 01	1.17*E* + 01	7.66*E* + 00	5.25*E* + 00	2.57*E* + 01	5.16*E* + 00	7.82*E* + 00	9.51*E* + 00
	Rank	2	6	1	4	10	11	12	8	7	9	5	3

cec07	AVE	9.65*E* + 02	9.61*E* + 02	9.82*E* + 02	8.70*E* + 02	1.28*E* + 03	1.01*E* + 03	1.41*E* + 03	1.28*E* + 03	1.46*E* + 03	1.34*E* + 03	1.10*E* + 03	9.53*E* + 02
	STD	5.18*E* + 01	4.31*E* + 01	5.08*E* + 01	2.71*E* + 01	9.97*E* + 01	1.38*E* + 02	4.69*E* + 01	7.66*E* + 01	4.41*E* + 02	3.45*E* + 01	4.92*E* + 01	6.10*E* + 01
	Rank	4	3	5	1	9	6	11	8	12	10	7	2

cec08	AVE	9.09*E* + 02	9.63*E* + 02	9.36*E* + 02	9.16*E* + 02	1.03*E* + 03	1.08*E* + 03	1.12*E* + 03	9.80*E* + 02	1.10*E* + 03	1.12*E* + 03	9.72*E* + 02	9.37*E* + 02
	STD	1.70*E* + 01	2.51*E* + 01	2.52*E* + 01	2.72*E* + 01	4.21*E* + 01	5.13*E* + 01	1.89*E* + 01	1.97*E* + 01	1.05*E* + 02	3.33*E* + 01	3.00*E* + 01	2.19*E* + 01
	Rank	1	5	3	2	8	9	12	7	10	11	6	4

cec09	AVE	3.65*E* + 03	4.30*E* + 03	3.52*E* + 03	4.01*E* + 03	1.18*E* + 04	1.01*E* + 04	9.98*E* + 03	8.20*E* + 03	1.29*E* + 04	5.92*E* + 03	6.66*E* + 03	4.42*E* + 03
	STD	1.42*E* + 03	6.54*E* + 02	1.15*E* + 03	2.79*E* + 03	3.19*E* + 03	2.01*E* + 03	1.40*E* + 03	1.06*E* + 03	5.39*E* + 03	4.74*E* + 02	1.57*E* + 03	2.31*E* + 03
	Rank	2	4	1	3	11	10	9	8	12	6	7	5

cec10	AVE	7.96*E* + 03	5.45*E* + 03	4.40*E* + 03	4.55*E* + 03	7.00*E* + 03	5.52*E* + 03	8.74*E* + 03	6.12*E* + 03	7.14*E* + 03	7.28*E* + 03	5.64*E* + 03	6.51*E* + 03
	STD	7.11*E* + 02	4.87*E* + 02	4.93*E* + 02	6.70*E* + 02	7.41*E* + 02	7.04*E* + 02	4.59*E* + 02	6.35*E* + 02	7.43*E* + 02	4.25*E* + 02	6.44*E* + 02	1.22*E* + 03
	Rank	11	3	1	2	8	4	12	6	9	10	5	7

cec11	AVE	1.21*E* + 03	4.12*E* + 03	2.40*E* + 03	1.35*E* + 03	7.35*E* + 03	1.89*E* + 03	1.14*E* + 04	1.31*E* + 03	2.47*E* + 04	1.15*E* + 04	2.50*E* + 03	1.21*E* + 03
	STD	4.19*E* + 01	9.40*E* + 02	2.14*E* + 03	4.61*E* + 01	3.28*E* + 03	7.22*E* + 02	3.55*E* + 03	4.51*E* + 01	1.76*E* + 04	3.38*E* + 03	8.16*E* + 02	3.52*E* + 01
	Rank	2	8	6	4	9	5	10	3	12	11	7	1

cec12	AVE	1.89*E* + 06	9.50*E* + 07	1.66*E* + 06	1.36*E* + 07	2.72*E* + 08	1.92*E* + 08	1.24*E* + 10	3.00*E* + 07	8.19*E* + 09	2.19*E* + 10	6.26*E* + 07	1.58*E* + 06
	STD	1.58*E* + 06	1.13*E* + 08	1.73*E* + 06	1.16*E* + 07	1.44*E* + 08	7.09*E* + 08	4.23*E* + 09	1.82*E* + 07	5.57*E* + 09	4.08*E* + 09	5.53*E* + 07	1.42*E* + 06
	Rank	3	7	2	4	9	8	11	5	10	12	6	1

cec13	AVE	8.20*E* + 03	3.39*E* + 04	3.37*E* + 05	1.26*E* + 05	2.14*E* + 06	1.15*E* + 05	5.58*E* + 09	5.61*E* + 05	8.50*E* + 09	2.32*E* + 10	1.46*E* + 06	5.90*E* + 03
	STD	7.39*E* + 03	1.03*E* + 04	8.82*E* + 05	5.71*E* + 04	1.69*E* + 06	6.57*E* + 04	4.20*E* + 09	2.09*E* + 05	5.02*E* + 09	8.00*E* + 09	2.51*E* + 06	4.64*E* + 03
	Rank	2	3	6	5	9	4	10	7	11	12	8	1

cec14	AVE	1.94*E* + 04	1.07*E* + 06	2.00*E* + 06	2.10*E* + 04	2.10*E* + 06	7.61*E* + 04	5.94*E* + 06	8.01*E* + 05	1.32*E* + 07	3.72*E* + 06	8.63*E* + 05	1.74*E* + 04
	STD	2.38*E* + 04	4.81*E* + 05	2.17*E* + 06	2.08*E* + 04	3.04*E* + 06	9.07*E* + 04	5.38*E* + 06	9.98*E* + 05	1.10*E* + 07	3.27*E* + 06	9.52*E* + 05	1.92*E* + 04
	Rank	2	7	8	3	9	4	11	5	12	10	6	1

cec15	AVE	3.99*E* + 03	1.65*E* + 04	8.85*E* + 03	4.94*E* + 04	2.69*E* + 06	8.04*E* + 04	4.81*E* + 08	9.60*E* + 04	1.67*E* + 09	4.65*E* + 08	1.10*E* + 05	4.57*E* + 03
	STD	2.76*E* + 03	5.06*E* + 03	9.96*E* + 03	3.84*E* + 04	4.51*E* + 06	8.43*E* + 04	3.44*E* + 08	8.92*E* + 04	1.26*E* + 09	4.38*E* + 08	5.92*E* + 04	2.27*E* + 03
	Rank	1	4	3	5	9	6	11	7	12	10	8	2

cec16	AVE	2.55*E* + 03	3.54*E* + 03	2.99*E* + 03	2.65*E* + 03	4.06*E* + 03	3.26*E* + 03	5.05*E* + 03	3.53*E* + 03	4.41*E* + 03	7.12*E* + 03	3.41*E* + 03	2.77*E* + 03
	STD	3.09*E* + 02	4.10*E* + 02	3.21*E* + 02	2.95*E* + 02	5.67*E* + 02	5.22*E* + 02	8.08*E* + 02	3.42*E* + 02	5.33*E* + 02	2.57*E* + 03	4.33*E* + 02	2.56*E* + 02
	Rank	1	8	4	2	9	5	11	7	10	12	6	3

cec17	AVE	2.05*E* + 03	2.77*E* + 03	2.58*E* + 03	2.08*E* + 03	2.72*E* + 03	2.60*E* + 03	3.89*E* + 03	2.69*E* + 03	4.04*E* + 03	9.59*E* + 03	2.48*E* + 03	2.02*E* + 03
	STD	1.31*E* + 02	2.66*E* + 02	2.63*E* + 02	1.24*E* + 02	3.10*E* + 02	2.61*E* + 02	1.08*E* + 03	2.65*E* + 02	8.24*E* + 02	1.40*E* + 04	3.02*E* + 02	1.67*E* + 02
	Rank	2	9	5	3	8	6	10	7	11	12	4	1

cec18	AVE	2.38*E* + 05	4.55*E* + 05	2.51*E* + 06	4.32*E* + 05	1.13*E* + 07	1.25*E* + 06	4.73*E* + 07	2.63*E* + 06	3.35*E* + 07	7.00*E* + 07	4.19*E* + 06	3.78*E* + 05
	STD	1.97*E* + 05	3.96*E* + 05	2.28*E* + 06	2.82*E* + 05	1.16*E* + 07	1.43*E* + 06	4.72*E* + 07	2.74*E* + 06	2.79*E* + 07	6.74*E* + 07	4.75*E* + 06	3.21*E* + 05
	Rank	1	4	6	3	9	5	11	7	10	12	8	2

cec19	AVE	5.65*E* + 03	1.63*E* + 05	9.55*E* + 03	1.13*E* + 06	1.10*E* + 07	3.09*E* + 06	8.91*E* + 08	1.22*E* + 06	1.48*E* + 09	6.38*E* + 08	2.13*E* + 06	4.90*E* + 03
	STD	3.26*E* + 03	1.93*E* + 05	5.79*E* + 03	7.32*E* + 05	9.76*E* + 06	2.12*E* + 06	6.30*E* + 08	1.22*E* + 06	1.63*E* + 09	4.82*E* + 08	1.97*E* + 06	2.09*E* + 03
	Rank	2	4	3	5	9	8	11	6	12	10	7	1

cec20	AVE	2.32*E* + 03	3.06*E* + 03	2.75*E* + 03	2.54*E* + 03	2.85*E* + 03	2.93*E* + 03	2.83*E* + 03	2.82*E* + 03	3.07*E* + 03	2.92*E* + 03	2.59*E* + 03	2.41*E* + 03
	STD	5.94*E* + 01	2.54*E* + 02	1.82*E* + 02	1.81*E* + 02	2.28*E* + 02	2.39*E* + 02	1.63*E* + 02	2.08*E* + 02	1.59*E* + 02	1.76*E* + 02	1.62*E* + 02	1.14*E* + 02
	Rank	1	11	5	3	8	10	7	6	12	9	4	2

cec21	AVE	2.41*E* + 03	2.62*E* + 03	2.47*E* + 03	2.41*E* + 03	2.65*E* + 03	2.65*E* + 03	2.72*E* + 03	2.57*E* + 03	2.62*E* + 03	2.72*E* + 03	2.47*E* + 03	2.40*E* + 03
	STD	2.20*E* + 01	3.23*E* + 01	2.73*E* + 01	2.91*E* + 01	5.90*E* + 01	8.14*E* + 01	7.78*E* + 01	5.72*E* + 01	1.08*E* + 02	4.20*E* + 01	4.77*E* + 01	1.86*E* + 01
	Rank	3	7	4	2	10	9	11	6	8	12	5	1

cec22	AVE	2.33*E* + 03	7.21*E* + 03	4.19*E* + 03	4.91*E* + 03	7.86*E* + 03	6.81*E* + 03	8.77*E* + 03	6.78*E* + 03	8.69*E* + 03	9.23*E* + 03	2.52*E* + 03	2.31*E* + 03
	STD	2.32*E* + 01	3.84*E* + 02	2.14*E* + 03	1.60*E* + 03	1.71*E* + 03	8.03*E* + 02	1.10*E* + 03	1.79*E* + 03	7.16*E* + 02	5.79*E* + 02	7.75*E* + 01	1.80*E* + 01
	Rank	2	8	4	5	9	7	11	6	10	12	3	1

cec23	AVE	2.81*E* + 03	3.80*E* + 03	2.83*E* + 03	2.76*E* + 03	3.11*E* + 03	3.24*E* + 03	3.48*E* + 03	3.22*E* + 03	2.99*E* + 03	3.52*E* + 03	2.96*E* + 03	2.78*E* + 03
	STD	5.06*E* + 01	1.55*E* + 02	4.98*E* + 01	2.99*E* + 01	7.35*E* + 01	9.98*E* + 01	1.59*E* + 02	1.19*E* + 02	6.72*E* + 01	1.63*E* + 02	5.99*E* + 01	3.59*E* + 01
	Rank	3	12	4	1	7	9	10	8	6	11	5	2

cec24	AVE	2.97*E* + 03	3.55*E* + 03	3.13*E* + 03	2.93*E* + 03	3.23*E* + 03	3.25*E* + 03	3.63*E* + 03	3.41*E* + 03	3.08*E* + 03	4.00*E* + 03	3.09*E* + 03	3.01*E* + 03
	STD	2.89*E* + 01	1.58*E* + 02	1.12*E* + 02	3.78*E* + 01	1.11*E* + 02	1.25*E* + 02	1.82*E* + 02	1.09*E* + 02	4.67*E* + 01	2.25*E* + 02	5.16*E* + 01	1.15*E* + 02
	Rank	2	10	6	1	7	8	11	9	4	12	5	3

cec25	AVE	2.93*E* + 03	2.99*E* + 03	2.99*E* + 03	2.90*E* + 03	3.09*E* + 03	2.93*E* + 03	5.64*E* + 03	2.94*E* + 03	5.14*E* + 03	7.89*E* + 03	3.00*E* + 03	2.91*E* + 03
	STD	2.58*E* + 01	2.68*E* + 01	3.46*E* + 01	1.80*E* + 01	5.19*E* + 01	4.53*E* + 01	6.17*E* + 02	2.49*E* + 01	2.27*E* + 03	6.65*E* + 02	2.42*E* + 01	1.55*E* + 01
	Rank	4	7	6	1	9	3	11	5	10	12	8	2

cec26	AVE	5.52*E* + 03	8.08*E* + 03	5.00*E* + 03	4.78*E* + 03	7.77*E* + 03	7.33*E* + 03	1.13*E* + 04	7.66*E* + 03	7.93*E* + 03	1.25*E* + 04	4.97*E* + 03	5.67*E* + 03
	STD	1.35*E* + 03	6.47*E* + 02	1.74*E* + 03	2.90*E* + 02	1.20*E* + 03	1.73*E* + 03	7.97*E* + 02	7.55*E* + 02	4.99*E* + 02	1.44*E* + 03	1.28*E* + 03	1.63*E* + 03
	Rank	4	10	3	1	8	6	11	7	9	12	2	5

cec27	AVE	3.30*E* + 03	5.13*E* + 03	3.27*E* + 03	3.23*E* + 03	3.46*E* + 03	3.36*E* + 03	4.05*E* + 03	3.50*E* + 03	3.35*E* + 03	4.79*E* + 03	3.39*E* + 03	3.20*E* + 03
	STD	2.79*E* + 01	3.90*E* + 02	2.52*E* + 01	1.44*E* + 01	1.16*E* + 02	1.66*E* + 02	3.78*E* + 02	1.15*E* + 02	3.92*E* + 01	6.27*E* + 02	7.24*E* + 01	1.15*E*-04
	Rank	4	12	3	2	8	6	10	9	5	11	7	1

cec28	AVE	3.35*E* + 03	3.58*E* + 03	3.32*E* + 03	3.25*E* + 03	3.60*E* + 03	3.36*E* + 03	6.94*E* + 03	3.33*E* + 03	6.63*E* + 03	8.71*E* + 03	3.47*E* + 03	3.31*E* + 03
	STD	4.36*E* + 01	2.04*E* + 02	5.87*E* + 01	4.26*E* + 01	9.05*E* + 01	3.54*E* + 02	8.10*E* + 02	3.02*E* + 01	2.61*E* + 02	8.66*E* + 02	8.74*E* + 01	2.49*E* + 01
	Rank	5	8	3	1	9	6	11	4	10	12	7	2

cec29	AVE	3.83*E* + 03	5.20*E* + 03	4.01*E* + 03	3.96*E* + 03	5.21*E* + 03	4.61*E* + 03	7.89*E* + 03	4.61*E* + 03	5.14*E* + 03	1.15*E* + 04	4.53*E* + 03	3.91*E* + 03
	STD	2.40*E* + 02	3.57*E* + 02	1.53*E* + 02	2.80*E* + 02	4.99*E* + 02	3.26*E* + 02	1.69*E* + 03	2.53*E* + 02	4.81*E* + 02	8.77*E* + 03	3.38*E* + 02	2.70*E* + 02
	Rank	1	9	4	3	10	6	11	7	8	12	5	2

cec30	AVE	1.38*E* + 04	2.60*E* + 06	1.01*E* + 06	4.24*E* + 06	4.55*E* + 07	6.65*E* + 06	1.06*E* + 09	4.85*E* + 06	1.32*E* + 09	3.02*E* + 09	1.14*E* + 07	1.19*E* + 04
	STD	6.07*E* + 03	1.37*E* + 06	2.78*E* + 06	3.53*E* + 06	4.24*E* + 07	5.50*E* + 06	1.26*E* + 09	2.36*E* + 06	1.15*E* + 09	1.54*E* + 09	6.51*E* + 06	4.76*E* + 03
	Rank	2	4	3	5	9	7	10	6	11	12	8	1
Mean rank		2.69	6.97	4.24	2.59	8.90	6.76	10.55	6.28	9.76	11.00	6.00	2.28
Final ranking		3	8	4	2	9	7	11	6	10	12	5	1

**Table 3:** The *p* value of the Wilcoxon rank-sum test on cec2017 test functions.

Functions	JS	GSA	CSO	MVO	WOA	GOA	LSO	HHO	ASO	AOA	AO
CEC01	1.18*E* − 02/−	1.00*E* + 00/=	1.91*E* − 06/−	4.14*E* − 02/+	1.91*E* − 06/−	1.15*E* − 01/=	1.91*E* − 06/−	1.91*E* − 06/−	1.91*E* − 06/−	1.91*E* − 06/−	1.91*E* − 06/−
CEC03	4.02*E* − 04/−	1.91*E* − 06/−	4.01*E* − 05/−	1.91*E* − 06/+	1.91*E* − 06/−	1.18*E* − 02	1.91*E* − 06/−	8.24*E* − 01/=	1.91*E* − 06/−	1.91*E* − 06/−	4.01*E* − 05/−
CEC04	8.24*E* − 01/=	2.58*E* − 03/−	4.14*E* − 02/−	2.58*E* − 03/+	1.91*E* − 06/−	8.24*E* − 01/=	1.91*E* − 06/−	1.15*E* − 01/=	1.91*E* − 06/−	1.91*E* − 06/−	1.91*E* − 06/−
CEC05	5.03*E* − 01/=	5.03*E* − 01/=	1.15*E* − 01/=	1.18*E* − 02/+	1.18*E* − 02/−	1.91*E* − 06/−	1.91*E* − 06/−	4.14*E* − 02/−	1.18*E* − 02/−	1.91*E* − 06/−	2.63*E* − 01/=
CEC06	1.00E + 00/=	1.91*E* − 06/−	1.91*E* − 06/+	1.00E + 00/=	1.91*E* − 06/−	1.91*E* − 06/−	1.91*E* − 06/−	1.91*E* − 06/−	1.91*E* − 06/−	1.91*E* − 06/−	1.91*E* − 06/−
CEC07	5.03*E* − 01/=	1.00E + 00/=	5.03*E* − 01/=	4.02*E* − 04/+	1.91*E* − 06/−	5.03*E* − 01/=	1.91*E* − 06/−	1.91*E* − 06/−	4.02*E* − 04/−	1.91*E* − 06/−	1.91*E* − 06/−
CEC08	1.15*E* − 01/=	4.14*E* − 02/−	5.03*E* − 01/=	4.14*E* − 02/+	1.91*E* − 06/−	1.91*E* − 06/−	1.91*E* − 06/−	4.14*E* − 02/−	4.01*E* − 05/−	1.91*E* − 06/−	5.03*E* − 01/=
CEC09	1.15*E* − 01/=	5.03*E* − 01/=	2.63*E* − 01/=	8.24*E* − 01/=	4.01*E* − 05/−	4.02*E* − 04/−	4.01*E* − 05/−	4.02*E* − 04/−	4.01*E* − 05/−	1.18*E* − 02/−	4.14*E* − 02/−
CEC10	1.15*E* − 01/=	4.02*E* − 04/+	4.01*E* − 05/+	1.91*E* − 06/+	8.24*E* − 01/=	4.02*E* − 04/+	4.01*E* − 05	1.18*E* − 02/+	1.00E + 00/=	2.63*E* − 01/=	2.58*E* − 03/+
CEC11	2.63*E* − 01/=	1.91*E* − 06/−	1.91*E* − 06/−	4.01*E* − 05/−	1.91*E* − 06/−	1.91*E* − 06/−	1.91*E* − 06/−	4.01*E* − 05/−	1.91*E* − 06/−	1.91*E* − 06/−	1.91*E* − 06/−
CEC12	5.03*E* − 01/=	1.91*E* − 06/−	8.24*E* − 01/=	1.91*E* − 06/−	1.91*E* − 06/−	1.91*E* − 06/−	1.91*E* − 06/−	1.91*E* − 06/−	1.91*E* − 06/−	1.91*E* − 06/−	1.91*E* − 06/−
CEC13	8.24*E* − 01/=	1.91*E* − 06/−	1.91*E* − 06/−	1.91*E* − 06/−	1.91*E* − 06/−	1.91*E* − 06/−	1.91*E* − 06/−	1.91*E* − 06/−	1.91*E* − 06/−	1.91*E* − 06/−	1.91*E* − 06/−
CEC14	8.24*E* − 01/=	1.91*E* − 06/−	1.91*E* − 06/−	1.15*E* − 01/=	1.91*E* − 06/−	4.14*E* − 02/−	1.91*E* − 06/−	1.91*E* − 06/−	1.91*E* − 06/−	1.91*E* − 06/−	1.91*E* − 06/−
CEC15	2.63*E* − 01/=	1.91*E* − 06/−	8.24*E* − 01/=	1.91*E* − 06/−	1.91*E* − 06/−	1.91*E* − 06/−	1.91*E* − 06/−	1.91*E* − 06/−	1.91*E* − 06/−	1.91*E* − 06/−	1.91*E* − 06/−
CEC16	2.63*E* − 01/=	4.02*E* − 04/−	4.14*E* − 02/−	5.03*E* − 01/=	1.91*E* − 06/−	1.18*E* − 02/−	1.91*E* − 06/−	1.91*E* − 06/−	1.91*E* − 06/−	1.91*E* − 06/−	4.01*E* − 05/−
CEC17	2.63*E* − 01/=	1.91*E* − 06/−	1.91*E* − 06/−	4.02*E* − 04/−	1.91*E* − 06/−	4.01*E* − 05/−	1.91*E* − 06/−	4.01*E* − 05/−	1.91*E* − 06/−	1.91*E* − 06/−	4.01*E* − 05/−
CEC18	8.24*E* − 01/=	4.14*E* − 02/−	4.02*E* − 04/−	1.18*E* − 02/−	4.01*E* − 05/−	4.02*E* − 04/−	1.91*E* − 06/−	2.58*E* − 03/−	1.91*E* − 06/−	1.91*E* − 06/−	4.01*E* − 05/−
CEC19	8.24*E* − 01/=	1.91*E* − 06/−	2.63*E* − 01/=	1.91*E* − 06/−	1.91*E* − 06/−	1.91*E* − 06/−	1.91*E* − 06/−	1.91*E* − 06/−	1.91*E* − 06/−	1.91*E* − 06/−	1.91*E* − 06/−
CEC20	5.03*E* − 01/=	1.91*E* − 06/−	1.18*E* − 02/−	5.03*E* − 01/=	1.91*E* − 06/−	4.01*E* − 05/−	1.91*E* − 06/−	4.01*E* − 05/−	1.91*E* − 06/−	1.91*E* − 06/−	2.58*E* − 03/−
CEC21	1.00E + 00/=	1.91*E* − 06/−	1.18*E* − 02/−	5.03*E* − 01/=	1.91*E* − 06/−	1.91*E* − 06/−	1.91*E* − 06/−	1.91*E* − 06/−	1.91*E* − 06/−	1.91*E* − 06/−	2.58*E* − 03/−
CEC22	1.15*E* − 01/=	1.91*E* − 06/−	4.01*E* − 05/−	4.01*E* − 05/−	1.91*E* − 06/−	1.91*E* − 06/−	1.91*E* − 06/−	1.91*E* − 06/−	1.91*E* − 06/−	1.91*E* − 06/−	1.91*E* − 06/−
CEC23	1.15*E* − 01/=	1.91*E* − 06/−	4.01*E* − 05/−	5.03*E* − 01/=	1.91*E* − 06/−	1.91*E* − 06/−	1.91*E* − 06/−	1.91*E* − 06/−	1.91*E* − 06/−	1.91*E* − 06/−	1.91*E* − 06/−
CEC24	1.00E + 00/=	4.01*E* − 05/−	2.63*E* − 01/=	8.24*E* − 01/=	2.63*E* − 01/=	1.15*E* − 01/=	1.91*E* − 06/−	1.91*E* − 06/−	2.63*E* − 01/=	1.91*E* − 06/−	5.03*E* − 01/=
CEC25	8.24*E* − 01/=	1.91*E* − 06/−	4.02*E* − 04/−	2.58*E* − 03/+	1.91*E* − 06/−	1.00E + 00/=	1.91*E* − 06/−	4.14*E* − 02/−	1.91*E* − 06/−	1.91*E* − 06/−	4.01*E* − 05/−
CEC26	8.24*E* − 01/=	1.91*E* − 06/−	8.24*E* − 01/=	1.15*E* − 01/=	1.91*E* − 06/−	2.58*E* − 03/−	1.91*E* − 06/−	4.02*E* − 04/−	4.02*E* − 04/−	1.91*E* − 06/−	8.24*E* − 01/=
CEC27	1.91*E* − 06/−	1.91*E* − 06/−	1.91*E* − 06/−	4.01*E* − 05/−	1.91*E* − 06/−	1.91*E* − 06/−	1.91*E* − 06/−	1.91*E* − 06/−	1.91*E* − 06/−	1.91*E* − 06/−	1.91*E* − 06/−
CEC28	2.63*E* − 01/=	1.91*E* − 06/−	1.00E + 00/=	4.01*E* − 05/+	1.91*E* − 06/−	4.14*E* − 02/−	1.91*E* − 06/−	4.14*E* − 02/−	1.91*E* − 06/−	1.91*E* − 06/−	1.91*E* − 06/−
CEC29	8.24*E* − 01/=	1.91*E* − 06/−	5.03*E* − 01/=	1.15*E* − 01/=	1.91*E* − 06/−	4.01*E* − 05/−	1.91*E* − 06/−	4.01*E* − 05/−	1.91*E* − 06/−	1.91*E* − 06/−	4.01*E* − 05/−
CEC30	1.00E + 00/=	1.91*E* − 06/−	1.15*E* − 01/=	1.91*E* − 06/−	1.91*E* − 06/−	1.91*E* − 06/−	1.91*E* − 06/−	1.91*E* − 06/−	1.91*E* − 06/−	1.91*E* − 06/−	1.91*E* − 06/−
+/−/=	0/26/3	1/4/24	2/12/15	9/10/10	0/2/27	1/5/23	0/0/29	1/2/26	0/2/27	0/1/28	1/4/24

**Table 4:** The number of function evaluations and execution times on cec2017 test functions.

Function	JS	GSA	CSO	MVO	WOA	GOA	LSO	HHO	ASO	AOA	AO	FOGJS
CEC01	2.7065	12.3922	6.0170	6.0348	2.2613	35.1929	1.9855	11.3714	20.9821	4.5290	11.6457	15.1768
CEC03	3.5131	12.2369	7.8752	5.3787	2.7771	35.5317	2.3484	10.1844	23.2933	4.9004	24.9698	16.0245
CEC04	2.6789	11.6298	5.9341	5.5321	2.0978	34.7803	1.6983	9.6181	22.0126	4.0862	10.4534	15.4520
CEC05	2.7505	11.7143	6.2998	5.7581	2.2609	35.0219	1.8799	11.9700	20.3889	4.8477	12.0491	14.5897
CEC06	5.0495	13.8682	12.9905	7.9945	4.5030	37.2236	4.1648	17.9729	26.0110	6.8288	17.8733	19.3789
CEC07	2.9198	11.9703	6.8966	5.9520	2.4580	35.2540	2.0748	12.3911	19.7669	4.9447	14.2293	14.9892
CEC08	2.8103	11.7521	6.5594	5.7971	2.3564	35.1671	1.9380	12.2690	20.5061	4.8929	12.2444	14.7867
CEC09	4.3631	13.1465	10.7201	7.3054	3.8079	38.6865	3.3674	14.1672	20.5218	4.8905	12.3131	18.0388
CEC10	5.0373	12.7053	9.6647	6.9376	3.4602	36.3130	3.2438	15.5772	29.0926	5.2186	13.1325	18.3623
CEC11	2.9487	11.8532	6.7883	5.1665	2.4030	35.3573	2.7793	10.4996	26.0504	4.4148	11.2691	15.3322
CEC12	3.6138	12.1908	7.9926	6.2011	2.7580	35.4513	2.6014	11.2374	26.3553	5.1620	11.8367	16.3858
CEC13	3.1011	11.8712	6.9422	5.8020	2.4297	35.2583	2.1285	10.7652	25.2373	4.4944	10.9107	15.3066
CEC14	4.2574	12.2911	8.1456	5.9011	2.8667	35.6623	2.5319	12.8246	26.5752	5.3377	12.6115	17.4529
CEC15	2.9989	11.7677	6.6305	5.6208	2.3407	35.2033	2.0122	10.3497	25.4023	4.3027	10.7015	15.3175
CEC16	3.6415	12.4632	7.8490	6.2351	2.7876	35.6124	2.3901	11.1907	26.7440	4.6606	11.5330	18.2657
CEC17	5.6991	14.3658	14.4855	8.4687	5.0384	37.9059	4.8134	16.2210	30.2044	6.7846	15.0185	22.2148
CEC18	3.3428	11.9307	7.0916	5.6584	2.4941	35.2894	2.0984	11.2186	25.6128	4.6969	11.3155	16.2910
CEC19	9.0490	17.8390	24.8333	11.8436	8.4414	41.2716	8.2289	39.8321	34.6625	15.8344	34.1780	28.8875
CEC20	6.7150	14.7896	15.6685	8.9579	5.4461	38.0852	5.2075	16.8818	30.0451	6.8492	15.5655	23.0113
CEC21	6.2876	15.0089	16.4831	9.1370	5.6521	38.3453	5.3954	19.7756	33.9069	8.1039	17.9104	22.4235
CEC22	7.4123	16.0146	19.7128	10.4190	6.8338	39.5789	6.6221	22.1463	31.5021	8.9067	20.0652	24.8958
CEC23	8.3140	16.7610	22.0370	11.2247	7.6950	40.2366	10.7281	23.7808	34.3246	9.9222	22.1497	27.9339
CEC24	8.0441	16.6313	21.4595	10.8171	7.3408	40.0270	8.5336	33.3528	35.4490	10.5150	23.8269	29.6309
CEC25	7.8619	16.7512	21.3756	10.8456	7.3697	39.9249	11.0523	29.1524	33.6303	9.3849	22.1971	25.8589
CEC26	9.8584	18.4609	26.9625	12.9988	9.4126	41.8311	12.4126	35.0726	35.9213	11.4311	26.3548	30.0543
CEC27	11.3057	19.5524	30.5458	14.0669	11.3285	42.9386	11.8015	38.1281	38.6731	12.6044	29.0552	46.5453
CEC28	9.8053	18.3297	26.6680	12.6377	10.6993	41.8145	11.3436	33.5285	35.7967	11.1153	25.8306	32.0283
CEC29	9.2615	17.8411	24.7765	11.9704	8.8397	41.0065	10.5643	29.9246	35.2396	9.2298	21.0481	29.3321
CEC30	12.7780	21.1413	35.0944	15.4022	12.1838	44.4547	14.7088	58.1867	40.5053	18.4674	39.2704	36.0754
NFFEs	30030	30000	90030	30000	30000	60000	31030	98461	30000	30030	60000	60030

**Table 5:** Results of FOGJS and other comparison algorithms on cec2019 test functions.

Function	Index	Algorithms											
		JS	PSO	DE	GBO	LSA	SOA	SSA	HGS	HBO	WHOA	AOA	FOGJS
Cec01	Best	1.00*E* + 00	8.24*E* + 03	4.08*E* + 04	1.00*E* + 00	3.08*E* + 03	1.00*E* + 00	1.00*E* + 00	1.00*E* + 00	2.72*E* + 05	1.00*E* + 00	3.06*E* + 07	1.00*E* + 00
	Worst	2.70*E* + 04	6.96*E* + 07	9.04*E* + 07	1.00*E* + 00	5.30*E* + 05	1.75*E* + 07	1.00*E* + 00	1.00*E* + 00	3.06*E* + 06	5.74*E* + 04	6.56*E* + 08	1.00*E* + 00
	Mean	1.86*E* + 03	5.30*E* + 06	1.96*E* + 07	1.00*E* + 00	1.05*E* + 05	1.83*E* + 06	1.00*E* + 00	1.00*E* + 00	1.50*E* + 06	1.04*E* + 04	1.88*E* + 08	1.00*E* + 00
	Std	6.05*E* + 03	1.60*E* + 07	2.88*E* + 07	8.16*E* − 13	1.27*E* + 05	4.13*E* + 06	5.95*E* − 15	0.00*E* + 00	8.95*E* + 05	1.83*E* + 04	1.46*E* + 08	0.00*E* + 00
	Rank	5	10	11	4	7	9	1	1	8	6	12	1

Cec02	Best	4.12*E* + 00	1.99*E* + 02	3.22*E* + 02	4.25*E* + 00	1.55*E* + 02	5.00*E* + 00	4.22*E* + 00	4.22*E* + 00	2.02*E* + 03	4.33*E* + 00	7.55*E* + 03	4.21*E* + 00
	Worst	3.10*E* + 01	7.17*E* + 03	1.35*E* + 04	5.00*E* + 00	5.12*E* + 02	4.45*E* + 03	5.00*E* + 00	2.48*E* + 01	5.73*E* + 03	5.73*E* + 00	2.15*E* + 04	4.28*E* + 00
	Mean	8.09*E* + 00	1.74*E* + 03	3.39*E* + 03	4.38*E* + 00	3.05*E* + 02	5.23*E* + 02	4.33*E* + 00	5.37*E* + 00	3.42*E* + 03	4.78*E* + 00	1.43*E* + 04	4.26*E* + 00
	Std	6.52*E* + 00	1.82*E* + 03	3.69*E* + 03	1.69*E* − 01	1.06*E* + 02	1.06*E* + 03	2.28*E* − 01	4.59*E* + 00	9.18*E* + 02	4.36*E* − 01	3.97*E* + 03	2.05*E* − 02
	Rank	6	9	10	3	7	8	2	5	11	4	12	1

Cec03	Best	1.09*E* + 00	1.82*E* + 00	4.61*E* + 00	1.41*E* + 00	1.00*E* + 00	4.00*E* + 00	1.45*E* + 00	1.41*E* + 00	4.48*E* + 00	1.00*E* + 00	4.49*E* + 00	1.41*E* + 00
	Worst	4.69*E* + 00	9.71*E* + 00	1.11*E* + 01	6.71*E* + 00	7.70*E* + 00	8.71*E* + 00	9.71*E* + 00	7.71*E* + 00	8.41*E* + 00	7.56*E* + 00	9.10*E* + 00	4.17*E* + 00
	Mean	2.90*E* + 00	5.25*E* + 00	8.79*E* + 00	1.67*E* + 00	2.40*E* + 00	7.25*E* + 00	5.63*E* + 00	3.83*E* + 00	7.13*E* + 00	2.63*E* + 00	7.32*E* + 00	2.68*E* + 00
	Std	1.01*E* + 00	2.37*E* + 00	1.63*E* + 00	1.19*E* + 00	2.18*E* + 00	1.94*E* + 00	2.66*E* + 00	2.44*E* + 00	1.08*E* + 00	1.82*E* + 00	1.19*E* + 00	8.85*E* − 01
	Rank	5	7	12	1	2	10	8	6	9	3	11	4

Cec04	Best	8.96*E* + 00	7.99*E* + 00	1.49*E* + 01	6.97*E* + 00	1.69*E* + 01	6.18*E* + 01	5.97*E* + 00	1.09*E* + 01	5.05*E* + 00	5.97*E* + 00	3.78*E* + 01	4.98*E* + 00
	Worst	4.68*E* + 01	7.06*E* + 01	6.32*E* + 01	4.78*E* + 01	8.26*E* + 01	1.24*E* + 02	9.75*E* + 01	3.78*E* + 01	1.89*E* + 01	3.03*E* + 01	1.09*E* + 02	5.17*E* + 01
	Mean	1.92*E* + 01	3.14*E* + 01	3.71*E* + 01	2.33*E* + 01	4.32*E* + 01	8.62*E* + 01	3.53*E* + 01	2.39*E* + 01	1.27*E* + 01	1.42*E* + 01	6.52*E* + 01	2.06*E* + 01
	Std	7.40*E* + 00	1.61*E* + 01	1.56*E* + 01	1.03*E* + 01	1.75*E* + 01	2.00*E* + 01	2.02*E* + 01	7.82*E* + 00	4.84*E* + 00	6.06*E* + 00	2.10*E* + 01	1.10*E* + 01
	Rank	3	7	9	5	10	12	8	6	1	2	11	4

Cec05	Best	1.02*E* + 00	1.16*E* + 00	1.02*E* + 00	1.02*E* + 00	1.02*E* + 00	2.78*E* + 01	1.05*E* + 00	1.02*E* + 00	1.00*E* + 00	1.02*E* + 00	5.75*E* + 01	1.02*E* + 00
	Worst	1.16*E* + 00	1.96*E* + 01	1.68*E* + 01	1.38*E* + 00	1.30*E* + 00	1.12*E* + 02	1.37*E* + 00	1.90*E* + 00	1.09*E* + 00	1.02*E* + 01	1.81*E* + 02	1.26*E* + 00
	Mean	1.08*E* + 00	5.00*E* + 00	2.53*E* + 00	1.15*E* + 00	1.13*E* + 00	6.56*E* + 01	1.14*E* + 00	1.19*E* + 00	1.02*E* + 00	1.53*E* + 00	1.28*E* + 02	1.08*E* + 00
	Std	3.35*E* − 02	5.42*E* + 00	3.67*E* + 00	7.61*E* − 02	6.11*E* − 02	2.18*E* + 01	7.29*E* − 02	1.96*E* − 01	2.48*E* − 02	2.05*E* + 00	3.32*E* + 01	5.97*E* − 02
	Rank	2	10	9	6	4	11	5	7	1	8	12	3

Cec06	Best	1.17*E* + 00	3.06*E* + 00	1.12*E* + 00	1.54*E* + 00	1.03*E* + 00	7.71*E* + 00	2.70*E* + 00	2.97*E* + 00	1.00*E* + 00	1.33*E* + 00	9.48*E* + 00	1.17*E* + 00
	Worst	4.61*E* + 00	9.39*E* + 00	9.49*E* + 00	7.52*E* + 00	7.60*E* + 00	1.36*E* + 01	7.76*E* + 00	8.46*E* + 00	1.64*E* + 00	8.41*E* + 00	1.43*E* + 01	4.16*E* + 00
	Mean	2.75*E* + 00	6.38*E* + 00	5.80*E* + 00	4.07*E* + 00	5.30*E* + 00	1.10*E* + 01	5.60*E* + 00	5.61*E* + 00	1.25*E* + 00	3.88*E* + 00	1.20*E* + 01	2.37*E* + 00
	Std	1.17*E* + 00	1.56*E* + 00	2.33*E* + 00	1.64*E* + 00	1.49*E* + 00	1.37*E* + 00	1.71*E* + 00	1.71*E* + 00	1.81*E* − 01	1.92*E* + 00	1.24*E* + 00	8.73*E* − 01
	Rank	3	10	9	5	6	11	7	8	1	4	12	2

Cec07	Best	3.60*E* + 02	6.08*E* + 02	3.82*E* + 02	5.35*E* + 02	1.35*E* + 02	1.31*E* + 03	4.35*E* + 02	3.39*E* + 02	4.71*E* + 02	3.23*E* + 02	7.59*E* + 02	4.19*E* + 02
	Worst	1.40*E* + 03	2.43*E* + 03	2.22*E* + 03	1.52*E* + 03	1.59*E* + 03	2.77*E* + 03	1.46*E* + 03	1.13*E* + 03	1.06*E* + 03	1.11*E* + 03	1.69*E* + 03	1.36*E* + 03
	Mean	8.82*E* + 02	1.19*E* + 03	1.37*E* + 03	9.56*E* + 02	9.63*E* + 02	2.24*E* + 03	8.42*E* + 02	7.05*E* + 02	7.69*E* + 02	6.51*E* + 02	1.36*E* + 03	8.59*E* + 02
	Std	2.66*E* + 02	4.41*E* + 02	5.07*E* + 02	2.49*E* + 02	3.77*E* + 02	4.19*E* + 02	2.85*E* + 02	2.29*E* + 02	1.72*E* + 02	2.00*E* + 02	2.69*E* + 02	2.47*E* + 02
	Rank	6	9	11	7	8	12	4	2	3	1	10	5

Cec08	Best	3.27*E* + 00	3.53*E* + 00	4.28*E* + 00	3.37*E* + 00	3.09*E* + 00	4.38*E* + 00	2.87*E* + 00	3.20*E* + 00	3.72*E* + 00	2.96*E* + 00	4.02*E* + 00	3.21*E* + 00
	Worst	4.27*E* + 00	4.85*E* + 00	5.43*E* + 00	4.58*E* + 00	4.53*E* + 00	5.19*E* + 00	4.96*E* + 00	4.80*E* + 00	4.44*E* + 00	4.47*E* + 00	5.50*E* + 00	4.14*E* + 00
	Mean	3.76*E* + 00	4.29*E* + 00	4.93*E* + 00	3.95*E* + 00	3.89*E* + 00	4.88*E* + 00	4.20*E* + 00	4.08*E* + 00	4.08*E* + 00	3.74*E* + 00	5.04*E* + 00	3.70*E* + 00
	Std	2.99*E* − 01	3.77*E* − 01	2.94*E* − 01	3.38*E* − 01	4.12*E* − 01	1.76*E* − 01	5.29*E* − 01	3.95*E* − 01	1.83*E* − 01	3.82*E* − 01	4.15*E* − 01	3.03*E* − 01
	Rank	3	9	11	5	4	10	8	7	6	2	12	1

Cec09	Best	1.12*E* + 00	1.06*E* + 00	1.12*E* + 00	1.06*E* + 00	1.12*E* + 00	1.30*E* + 00	1.15*E* + 00	1.13*E* + 00	1.12*E* + 00	1.07*E* + 00	2.91*E* + 00	1.14*E* + 00
	Worst	1.37*E* + 00	1.44*E* + 00	1.84*E* + 00	1.45*E* + 00	1.50*E* + 00	5.23*E* + 00	1.72*E* + 00	1.63*E* + 00	1.27*E* + 00	1.42*E* + 00	5.00*E* + 00	1.35*E* + 00
	Mean	1.23*E* + 00	1.24*E* + 00	1.35*E* + 00	1.21*E* + 00	1.29*E* + 00	3.25*E* + 00	1.36*E* + 00	1.31*E* + 00	1.21*E* + 00	1.22*E* + 00	3.78*E* + 00	1.28*E* + 00
	Std	6.64*E* − 02	1.11*E* − 01	1.71*E* − 01	1.01*E* − 01	1.07*E* − 01	1.04*E* + 00	1.92*E* − 01	1.21*E* − 01	3.25*E* − 02	1.06*E* − 01	4.95*E* − 01	5.14*E* − 02
	Rank	4	5	9	2	7	11	10	8	1	3	12	6

Cec10	Best	5.66*E* + 00	2.10*E* + 01	2.13*E* + 01	2.16*E* + 00	2.10*E* + 01	2.16*E* + 01	2.10*E* + 01	2.10*E* + 01	2.11*E* + 01	2.10*E* + 01	2.10*E* + 01	3.01*E* + 00
	Worst	2.15*E* + 01	2.14*E* + 01	2.20*E* + 01	2.14*E* + 01	2.15*E* + 01	2.19*E* + 01	2.13*E* + 01	2.11*E* + 01	2.13*E* + 01	2.11*E* + 01	2.10*E* + 01	2.15*E* + 01
	Mean	2.05*E* + 01	2.12*E* + 01	2.16*E* + 01	2.03*E* + 01	2.12*E* + 01	2.17*E* + 01	2.10*E* + 01	2.10*E* + 01	2.12*E* + 01	2.10*E* + 01	2.10*E* + 01	1.89*E* + 01
	Std	3.52*E* + 00	1.41*E* − 01	1.97*E* − 01	4.26*E* + 00	1.63*E* − 01	7.66*E* − 02	8.48*E* − 02	2.59*E* − 02	4.91*E* − 02	1.63*E* − 02	3.66*E* − 03	6.03*E* + 00
	Rank	3	10	11	2	8	12	7	6	9	5	4	1

Mean rank		4	8.6	10.2	4	6.3	10.6	6	5.6	5	3.8	10.8	2.8
Final ranking		3	9	10	3	8	11	7	6	5	2	12	1

**Table 6:** The *p* value of the Wilcoxon rank-sum test on cec2019 test functions.

Functions	JS	PSO	D*E*	GBO	LSA	SOA	SSA	HGS	HBO	WHOA	AOA
CEC01	1.91*E* − 06/−	8.01*E* − 09/−	8.01*E* − 09/−	NaN/=	1.91*E* − 06/−	7.63*E* − 06/−	1.00*E* + 00/=	NaN/=	8.01*E* − 09/−	7.63*E* − 06/−	1.91*E* − 06/−
CEC02	1.91*E* − 06/−	6.80*E* − 08/−	6.80*E* − 08/−	1.41*E* − 05/−	1.91*E* − 06/−	1.91*E* − 06/−	2.63*E* − 01/=	3.23*E* − 01/=	6.80*E* − 08/−	1.91*E* − 06/−	1.91*E* − 06/−
CEC03	1.15*E* − 01/−	1.66*E* − 07/−	6.80*E* − 08/−	4.36*E* − 07/+	1.18*E* − 02/+	1.91*E* − 06/−	4.14*E* − 02/−	5.07*E* − 01/=	6.80*E* − 08/−	5.03*E* − 01/=	1.91*E* − 06/−
CEC04	5.03*E* − 01/=	1.44*E* − 02/−	3.38*E* − 04/−	2.98*E* − 01/=	4.02*E* − 04/−	1.91*E* − 06/−	1.18*E* − 02/−	6.55*E* − 01/=	1.33*E* − 02/+	2.63*E* − 01/=	1.91*E* − 06/−
CEC05	4.14*E* − 02/+	2.22*E* − 07/−	3.38*E* − 04/−	6.22*E* − 04/−	4.14*E* − 02/−	1.91*E* − 06/−	4.14*E* − 02/−	3.75*E* − 04/−	2.79*E* − 03/+	8.24*E* − 01/=	1.91*E* − 06/−
CEC06	2.63*E* − 01/=	6.92*E* − 07/−	1.58*E* − 06/−	6.22*E* − 04/−	4.01*E* − 05/−	1.91*E* − 06/−	4.02*E* − 04/−	1.80*E* − 06/−	7.58*E* − 06/+	1.18*E* − 02/−	1.91*E* − 06/−
CEC07	8.24*E* − 01/=	1.23*E* − 02/−	2.04*E* − 05/−	2.39*E* − 01/=	2.63*E* − 01/=	1.91*E* − 06/−	2.63*E* − 01/=	6.79*E* − 02/=	8.39*E* − 01/=	1.18*E* − 02/+	4.02*E* − 04/−
CEC08	2.63*E* − 01/=	3.75*E* − 04/−	6.80*E* − 08/−	4.39*E* − 02/−	5.03*E* − 01/=	1.91*E* − 06/−	2.58*E* − 03/−	1.33*E* − 02/−	2.47*E* − 04/−	2.63*E* − 01/=	1.91*E* − 06/−
CEC09	5.03*E* − 01/=	5.25*E* − 01/=	6.55*E* − 01/−	1.14*E* − 02/+	1.00*E* + 00/=	1.91*E* − 06/−	8.24*E* − 01/=	4.09*E* − 01/=	4.70*E* − 03/+	1.15*E* − 01/=	1.91*E* − 06/−
CEC10	4.14*E* − 02/−	5.98*E* − 01/=	9.28*E* − 05/−	4.25*E* − 01/=	8.24*E* − 01/=	1.91*E* − 06/−	8.24*E* − 01/=	7.11*E* − 03/−	7.64*E* − 02/=	4.14*E* − 02/−	4.14*E* − 02/−
+/=/−	1/5/4	0/2/8	0/0/10	2/3/5	1/4/5	0/0/10	0/5/5	0/6/4	4/2/4	1/5/4	0/0/10

**Table 7:** The number of function evaluations and execution times on cec2019 test functions.

Function	JS	PSO	DE	GBO	LSA	SOA	SSA	HGS	HBO	WHOA	AOA	FOGJS
CEC01	3.6200	2.8114	6.0888	15.7707	30.2908	4.3671	7.5269	4.3323	4.6441	13.9102	3.4599	15.6979
CEC02	2.1869	1.3686	6.0189	14.4759	47.7168	4.2256	5.3505	2.7221	3.7760	12.2332	2.2003	13.3965
CEC03	2.8174	1.3118	6.3777	15.5053	52.3774	4.5143	5.4665	2.7589	3.7545	12.3701	2.2264	13.4125
CEC04	2.5652	1.5433	4.9453	14.2501	36.4910	3.2141	5.7330	2.6113	3.2024	12.3221	2.1680	13.8916
CEC05	2.5422	1.5809	4.9875	14.3659	34.9856	3.2794	5.7593	2.6728	3.2467	12.3997	2.2298	13.9198
CEC06	20.3736	18.8581	22.2178	33.9569	74.9322	20.5988	34.6231	19.9502	20.2233	30.5913	19.6429	49.0128
CEC07	3.2563	1.7084	5.1264	14.5384	36.4959	3.3727	6.0191	2.7732	3.4223	12.5532	2.3344	15.2189
CEC08	2.7577	1.5725	4.9911	14.4529	30.2979	3.2464	5.7523	2.6618	3.2323	12.4473	2.1979	14.4652
CEC09	2.1947	1.3554	4.7838	14.1492	37.5057	3.0529	5.2918	2.4728	3.0199	11.8400	2.0393	13.3624
CEC10	3.2142	1.5874	4.9943	14.4306	41.9134	3.2798	5.8652	2.6894	3.2357	12.4172	2.2075	15.1973
NFFEs	30030	30030	30030	30030	107584	30030	90030	30000	30030	150030	30030	60030

**Table 8:** Result of the predicted model based on different algorithms.

	FOGJS	JS	AO	SCA	GWO	RSO	SOA	DE	PSO
Best	**10.3858**	10.3859	10.3893	10.3895	10.3859	10.3860	10.3888	10.3859	**10.3858**
Mean	**10.3860**	10.3873	10.4338	10.4149	10.3974	10.4267	10.4174	10.3877	10.3970
Worst	**10.3865**	10.3909	10.6427	10.4926	10.4329	10.5582	10.4819	10.3940	10.4117
Std	**2.1697*E* − 04**	1.6785*E* − 03	7.4951*E* − 02	3.0414*E* − 02	1.4576*E* − 02	5.6484*E* − 02	3.1718*E* − 02	2.4713*E* − 03	8.7028*E* − 03

**Table 9:** Evaluation indicators.

Measure indicators	Formula
Mean absolute error (MAE)	$\left(1/n\right)\sum_{k=1}^{n}\left|{\hat{z}}^{\left(0\right)}\left(k\right)-z^{\left(0\right)}\left(k\right)\right|$
Mean absolute percentage error (MAPE)	$\left(1/n\right)\sum_{k=1}^{n}\left|{\hat{z}}^{\left(0\right)}\left(k\right)-z^{\left(0\right)}\left(k\right)\right|\times 100\%$
Mean square error (MSE)	$\left(1/n\right){\sum_{k=1}^{n}\left({\hat{z}}^{\left(0\right)}\left(k\right)-z^{\left(0\right)}\left(k\right)\right)}^{2}$
Root mean square percentage error (RMSPE)	$\sqrt{\left(1/n\right)\sum_{k=1}^{n}{\left({\hat{z}}^{\left(0\right)}\left(k\right)-z^{\left(0\right)}\left(k\right)/z^{\left(0\right)}\left(k\right)\right)}^{2}}\times 100\%$

**Table 10:** Fitting results of different forecast models.

Years	Actual income	GM	DGM	TRGM	FANGBM	FTDGM	DFTDGM	TDFTDGM
1989	433.67	434.00	434.00	434.00	434.00	434.00	434.00	434.00
1990	530.00	306.97	311.02	569.77	483.14	537.18	483.23	542.11
1991	533.96	347.14	351.70	635.64	537.88	640.47	538.04	534.00
1992	558.79	392.57	397.71	709.11	598.85	743.90	599.08	648.42
1993	652.99	443.95	449.73	791.08	666.77	847.48	667.03	657.57
1994	804.84	502.04	508.56	882.53	742.44	951.26	742.70	786.08
1995	962.89	567.75	575.08	984.54	826.76	1055.29	826.94	816.24
1996	1165.10	642.04	650.30	1098.35	920.71	1159.60	920.75	963.04
1997	1273.30	726.07	735.36	1225.31	1025.41	1264.27	1025.19	1018.92
1998	1415.08	821.08	831.55	1366.95	1142.11	1369.37	1141.48	1189.29
1999	1474.96	928.53	940.32	1524.96	1272.19	1475.00	1270.96	1294.69
2000	1471.67	1050.05	1063.32	1701.24	1417.21	1581.27	1415.13	1477.34
2001	1529.11	1187.46	1202.40	1897.89	1578.89	1688.31	1575.66	1585.97
2002	1648.04	1342.86	1359.68	2117.28	1759.19	1796.31	1754.39	1842.90
2003	1741.11	1518.60	1537.53	2362.02	1960.25	1905.46	1953.40	2035.64
2004	1952.57	1717.33	1738.65	2635.06	2184.52	2016.01	2174.98	2305.63
2005	2161.68	1942.07	1966.07	2939.66	2434.71	2128.27	2421.69	2522.53
2006	2396.33	2196.22	2223.24	3279.46	2713.85	2242.60	2696.39	2890.23
2007	2824.05	2483.63	2514.05	3658.55	3025.34	2359.47	3002.26	3217.49
2008	3373.46	2808.65	2842.90	4081.46	3373.00	2479.41	3342.81	3627.64
2009	3722.07	3176.21	3214.76	4553.25	3761.09	2603.10	3722.00	4011.96
2010	4477.21	3591.86	3635.26	5079.58	4194.40	2731.35	4144.20	4520.87
2011	5483.79	4061.92	4110.77	5666.76	4678.29	2865.13	4614.29	5092.62
2012	6285.00	4593.48	4648.48	6321.80	5218.78	3005.67	5137.71	5725.99
2013	7092.20	5194.61	5256.51	7052.56	5822.62	3154.42	5720.50	6370.73

**Table 11:** Fitting error of different forecast models.

	GM	DGM	TRGM	FANGBM	FTDGM	DFTDGM	TDFTDGM
MAE	519	499	320	248	627	256	**221**
MAPE (%)	25.606	24.725	16.212	**9.696**	17.258	9.763	9.873
MSE	488381	454256	200193	163109	1546543	185217	**85490**
RMSPE (%)	28.488	27.717	20.539	**11.653**	24.240	11.796	12.034

**Table 12:** Predicted results of different forecast models.

Years	Actual income	GM	DGM	TRGM	FANGBM	FTDGM	DFTDGM	TDFTDGM
2014	7932.21	5874.41	5944.09	7867.80	6497.38	3313.16	6369.39	7232.41
2015	8689.00	6643.17	6721.60	8777.27	7251.58	3484.06	7091.90	8057.86
2016	9396.00	7512.53	7600.81	9791.88	8094.78	3669.75	7896.36	9045.05
2017	10264.51	8495.67	8595.03	10923.76	9037.73	3873.45	8792.07	10096.47
2018	11213.00	9607.46	9719.29	12186.49	10092.53	4099.05	9789.38	11331.47
2019	12326.00	10864.75	10990.61	13595.18	11272.79	4351.32	10899.83	12737.23
2020	13316.00	12286.57	12428.23	15166.70	12593.82	4636.02	12136.24	14283.60

**Table 13:** Predicted error of different forecast models.

	GM	DGM	TRGM	FANGBM	FTDGM	DFTDGM	TDFTDGM
MAE	1693	1591	757	1185	6530	1452	**478**
MAPE (%)	17.239	16.271	6.477	12.056	62.095	14.502	**4.731**
MSE	2981279	2662247	940980	1458475	44515496	2123232	**308408**
RMSPE (%)	18.250	17.361	7.885	12.749	62.140	14.929	**5.507**

**Table 14:** The predicted results from 2021 to 2025 based on different forecast models.

Years	GM	DGM	TRGM	FANGBM	FTDGM	DFTDGM	TDFTDGM
2021	13894.46	14053.89	16919.89	14072.94	4960.21	13512.89	14782.68
2022	15712.77	15892.20	18875.73	15729.55	5332.43	15045.71	16450.74
2023	17769.04	17970.96	21057.66	17585.65	5763.11	16752.40	18307.02
2024	20094.40	20321.64	23491.80	19666.03	6264.93	18652.68	20372.76
2025	22724.07	22979.79	26207.32	21998.72	6853.30	20768.53	22671.59

## Data Availability

All data generated or analyzed during this study are included in this published article (and its supplementary information files).

## Supplementary Materials

Supplementary Materials The Matlab Code of the proposed FOGJS.
